# Single- versus Dual-Targeted Nanoparticles with Folic Acid and Biotin for Anticancer Drug Delivery

**DOI:** 10.3390/pharmaceutics13030326

**Published:** 2021-03-03

**Authors:** Magdalena Jurczyk, Katarzyna Jelonek, Monika Musiał-Kulik, Artur Beberok, Dorota Wrześniok, Janusz Kasperczyk

**Affiliations:** 1 Centre of Polymer and Carbon Materials, Polish Academy of Sciences, 41-819 Zabrze, Poland; d200967@365.sum.edu.pl (M.J.); mmusial@cmpw-pan.edu.pl (M.M.-K.); janusz.kasperczyk@sum.edu.pl (J.K.); 2 Department of Pharmaceutical Chemistry, Faculty of Pharmaceutical Sciences in Sosnowiec, Medical University of Silesia, 41-200 Sosnowiec, Poland; abeberok@sum.edu.pl (A.B.); dwrzesniok@sum.edu.pl (D.W.); 3 Department of Biopharmacy, Faculty of Pharmaceutical Sciences in Sosnowiec, Medical University of Silesia, 41-200 Sosnowiec, Poland

**Keywords:** targeted delivery, dual-targeted, nanoparticles, anticancer drugs, folic acid, biotin, active targeting, drug delivery, vitamin, ligand

## Abstract

Cancer is one of the major causes of death worldwide and its treatment remains very challenging. The effectiveness of cancer therapy significantly depends upon tumour-specific delivery of the drug. Nanoparticle drug delivery systems have been developed to avoid the side effects of the conventional chemotherapy. However, according to the most recent recommendations, future nanomedicine should be focused mainly on active targeting of nanocarriers based on ligand-receptor recognition, which may show better efficacy than passive targeting in human cancer therapy. Nevertheless, the efficacy of single-ligand nanomedicines is still limited due to the complexity of the tumour microenvironment. Thus, the NPs are improved toward an additional functionality, e.g., pH-sensitivity (advanced single-targeted NPs). Moreover, dual-targeted nanoparticles which contain two different types of targeting agents on the same drug delivery system are developed. The advanced single-targeted NPs and dual-targeted nanocarriers present superior properties related to cell selectivity, cellular uptake and cytotoxicity toward cancer cells than conventional drug, non-targeted systems and single-targeted systems without additional functionality. Folic acid and biotin are used as targeting ligands for cancer chemotherapy, since they are available, inexpensive, nontoxic, nonimmunogenic and easy to modify. These ligands are used in both, single- and dual-targeted systems although the latter are still a novel approach. This review presents the recent achievements in the development of single- or dual-targeted nanoparticles for anticancer drug delivery.

## 1. Introduction

According to the World Cancer Report [1], cancer is the first or second leading cause of premature death (i.e., at ages 30–69 years) in 134 of 183 countries and it ranks third or fourth in an additional 45 countries. Therefore, cancer treatment represents one of the most crucial issues in clinical management [2]. First-line therapy of solid tumours is based on surgery, radiotherapy and/or chemotherapy [3]. For metastasized tumours, or for lesions, which cannot be removed surgically, chemotherapy is among the very few treatment options available. The serious problem of intravenous systemic chemotherapy is the unspecific targeting to the tumour and difficulties to achieve therapeutic levels of drug within or adjacent to the tumour. For example, in the case of intravenously infused paclitaxel (Ptx), less than 0.5% of the total dose is locally available within the tumour. Furthermore, significant concentrations of drug frequently accumulate in healthy tissue, leading to severe side effects and dose-limiting toxicity [4]. Different strategies have been tried to develop novel tumour-specific delivery systems for chemotherapeutics to reduce toxicity and recent progress in nanomedicine have created an opportunity for the development of more potent and tumour-targeted dosage forms [5]. So far, various kinds of nanomedicines such as antibody-drug conjugates (ADCs), drug conjugates and nanocarriers for cancer therapy have been approved by the US Food and Drug Administration (FDA) and European Medicines Agencies (EMA) [6]. Liposomal doxorubicin (Doxil™/Caelyx™) was the first anti-cancer nanomedicine approved by the FDA in 1995 and it achieved a nearly 300-fold increase in area under the curve, relative to free doxorubicin [7]. Liposomes are spherical structures composed of phospholipid bilayers and cholesterol that enclose centre space that can carry small drug molecules and large macromolecules like DNA. They characterize a large cargo space and capability to simultaneously deliver both, hydrophilic and hydrophobic agents. Liposomes also provide longer circulation time than free drug and can be easily modified to obtain the expected therapeutic effect [8]. Apart from surface modification for achieving the active targeting, the liposomes may also respond to the specific properties of the cancer cell environment to release anti-cancer drugs under well-defined conditions, e.g., pH, ultrasounds, magnetic field exposure, light, enzymes, thereby reducing systemic toxicity to healthy cells [9]. An example of stimuli-responsive liposomes are magnetoliposomes, which possess a magnetic core surrounded by lipid bilayer. The magnetoliposomes may be excited by magnetic radiation that cause local hyperthermia within the tumor leading to the cancer cell death. Such transport systems, in addition, to their chemotherapeutic properties, can also be used in cancer diagnostics (e.g., with the use of MRI) and may be promising in the future cancer therapy [10,11]. However, apart from liposomes, also other kinds of nanoparticles are already studied for anticancer drug delivery, e.g., dendrimers or polymeric micelles. Dendrimers have a well-defined macromolecular structure, spherical geometry and abundant functional groups on the surface that can be modified or physically changed for nontoxicity, enhanced efficiency and specific cargo abilities [12]. Research studies consider dendrimers as delivery systems for drugs, genes and contrast agents [13]. There are few different types of compounds used for preparation of dendrimers, e.g., poly(propylene imine) (PPI), poly(L-lysine), poly(amidoamine) (PAMAM), PAMAM-organosilicon (PAMAMOS). Dendrimers, in comparison to other polymeric delivery systems, have many specific advantages: (1) the well-known, predictable size, macromolecular weight and structure, which results in desirable abilities to deliver active agent, as well as the option to choose an appropriate structure with expected properties; (2) controllable size, lipophilicity and ability to cross cell walls; (3) adjustability by many compounds of their terminal ends, resulting in a change of the dendrimers properties, toxicity level, target point, etc. [14].

Polymeric micelles are small core-shell structures, formed by self-assembly of amphiphilic block copolymers that have the ability to increase drug solubility and reduce toxicity [15]. The hydrophobic core is surrounded by a hydrophilic shell. The most popular polymer forming the outer shell is poly(ethylene glycol) (PEG) due to its hydrophilicity and biocompatibility. Poly(lactide) (PLA) and poly(ε-caprolactone) (PCL) are one of the most commonly used hydrophobic blocks of the amphiphilic polymers because they are biocompatible and biodegradable [16]. The size of polymer micelles between 50–200 nm support long-term circulation and avoiding capturing by the reticuloendothelial system. Compared to surfactant micelles, block copolymer-based micelles are characterized by higher stability and larger versatility for controlling micellar structure and functionality by choices of polymer composition, architecture, molecular weight and monomer chemistry [17]. Moreover, surface modification enables enhanced tissue penetration and targeting properties [18,19,20].

It has been demonstrated that substantial intra- and intertumoural variability is present in the tumour cells and the tumour microenvironment that results in the heterogeneity of molecular, pathologic and clinical features of each tumour type. In this aspect, the nanoparticle design plays a significant role in influencing tumour targeting [5].

## 2. Active Targeting of Nanoparticles

Passive targeting associated with the enhanced permeability and retention (EPR) effect was proposed as the major underlying mechanism for nanomedicine-based cancer therapy. However, more and more studies have revealed that although the EPR effect, present in animals like mice, plays a less important role in humans due to tumour heterogeneity or lack of fenestrations in the tumour endothelium [6]. Therefore, the most recent reports indicate that future nanomedicine may require new design principles toward an active targeting of nanocarriers [3,6,21,22].

In order to specifically target and eradicate cancer cells, there is a requirement for precise distinguishing target cells (tumour cells) from non-target cells and development of smart drug delivery platforms [23]. Active-targeting based on ligand-receptor recognition may show better efficacy than passive targeting in human cancer therapy and several active-targeting nanomedicines have already progressed into clinical trials [24]. Targeted drug delivery systems can be also useful to overcome the acquired multidrug resistance (MDR), which is supposed to be caused by overexpression of superfamily of ATP-binding cassette (ABC) proteins, e.g., P-glycoprotein (P-gp) and multi resistance-associated protein (MRP) that result in enhanced cellular efflux [25,26]. 

In the past decade, several strategies for receptor mediated endocytosis have been developed to enhance tumour cell uptake of drug-loaded nanoparticles. A variety of small molecules such as folic acid (FA) and biotin (BIO) (Figure 1) have been used as targeting ligands for cancer chemotherapy, because they are readily available, inexpensive, nontoxic, nonimmunogenic and easy to modify [27]. Based on the overexpression of specific receptors on tumour cells, active targeting nanomedicines may efficiently deliver drugs into tumour cells via receptor-mediated endocytosis, so the targeting effect is affected by the receptor expression. The folate and biotin as a low-molecular-weight vitamins play essential roles in cell survival and bind to the respective receptors with high affinity. The folate and biotin receptors are up-regulated in various carcinomas while being expressed at low levels in normal cells and tissues, thereby minimizing the potential off-target toxicities [28].

However, since the receptors (surface markers) of tumour cells change dynamically with tumour progression [29], the multiple ligand-coated nanostructures have been found to improve the identification of the tumour cells [6,23].

## 3. Folic Acid—Targeted Nanoparticles

### 3.1. Folic Acid as a Targeting Ligand

Recent studies show the great potential of folic acid-targeted drug delivery systems [13]. The FA (B9 vitamin) is necessary for the synthesis of purines and thymidine—the crucial nucleic acids components. Folate receptors (FRs) are membrane glycoproteins that uptake folians through endocytosis. There are three different subforms of FRs—Frα, Frβ and Frγ—identified in human tissues. An increased folic requirement in fast proliferating cells, such as cancer tissues, cause a higher expression level of FRα compared to healthy cells [30]. Thus, FA receptors are overexpressed in human carcinomas including breast, ovary, endometrium, kidney, lung, head and neck, brain, colon and myeloid cancers, while only minimally distributed in normal tissues [31,32,33,34,35]. The abundance of folate receptors per cell varies dramatically, from approximately ~3 × 10^5^ in KB oral carcinoma cells and about 10^4^ in C6 glioma cells down to undetectable in E9 chick cortical cells [36]. The expression of the folate receptor alpha (FRα) is significantly increased in patients with triple-negative breast cancer and is therefore, a potential biomarker and therapeutic target [37,38,39]. The FR is also highly expressed in bone metastatic cells and osteoclasts [40], being an attractive target for bone-related cancers. Thus, using the FRs as a target for drug delivery systems is based on the specific characteristic of these receptor types: much higher overexpression on tumours cells (100–300×), rapid receptor recirculation after cell internalization and exposition on a cell surface without releasing to circulation [13,41]. Moreover, small molecules like folic acid present advantages over peptides or antibodies as targeting ligands, e.g., improved stability during storage, increased stability in acidic or basic media and better resistance to high temperature. Folic acid carries no risk of toxicity or immune reactions, offers unlimited availability and low cost as well as low immunogenicity. As a targeting ligand FA is also easy to scale-up for clinical applications and facile chemical modification [13,41]. Therefore, the FR-targeted drug delivery for different cell types or specific organs can potentially maximize therapeutic efficacy while minimizing side effects.

### 3.2. Examples of Folic Acid-Targeted Nanoparticles

The currently developed FA-targeted drug delivery systems include various kinds of nanoparticles, e.g., liposomes, micelles, carbon nanotubes, nanorods, core-shell quantum dots, nanospheres, mesoporous nanoparticles and dendrimers (Table 1, Figure 2). The NP have been analysed for achieving an effective antitumour effect by several strategies: single drug delivery [42,43,44,45,46], co-delivery of more than one drug [47,48,49], co-delivery of drug and gene [50,51,52,53], phototherapy [54,55,56], systems combining cancer treatment and diagnosis [57,58,59,60,61] and gene delivery [53,62]. Some drug delivery systems use magnetic ions [63,64,65] or gold nanoparticles [66].

#### 3.2.1. Drug Delivery Application

##### Single-Drug Delivery

Targeted properties of liposomes can be achieved by conjugation with ligands. Although the mono-targeting ligand can promote the binding and internalization of liposomes into the cancer cells, only a few liposomes with high targeting efficiency have been developed so far, because the traditional mono-branched ligand modified liposomes generally fail to deliver an adequate therapeutic payload [85]. Studies showed that functionalization with folic acid resulted in reduced drug uptake into noncancerous cells, higher cytotoxicity to cancer cells with FR overexpression, better tumour shrinkage efficiency, prolonged mice survival time, reduced mice weight loss and much lower toxicity compared to free drug or not targeted drug-loaded liposomes [67,68,69,70,71,72]. Folic acid conjugated liposomes may also be applied as a tumour imaging tool that enables to enhance diagnostics of small tumours [86,87,88].

There are extensive studies on FA-targeted micelles. Varshosaz et al. synthesized folic acid targeted micelles of Synperonic PE/F 127-cholesteryl hemisuccinate (PF127-Chol) loaded with docetaxel. In vitro studies exhibited the high drug encapsulation efficiency of 99.6% and superior cytotoxicity and cellular uptake in comparison to not-targeted micelles and free drug. Moreover, a reduction in tumour volume was observed in mice bearing melanoma [78]. pH-sensitive and folic acid-targeted mixed micelles were developed from a mixture of poly(ethylene glycol)/methyl ether-poly(histidine) (MPEG-PHIS) and folic acid-poly(ethylene glycol)-(+)-α-tocopherol (FA-PEG-VE). These micelles presented high cytotoxicity and destabilisation in the acid environment of endosomes, which caused the release of paclitaxel. The rate of sarcoma tumour inhibition in female Kunming mice was 85.97% [19]. Recent studies evaluated the drug delivery system encapsulated with doxorubicin, which was composed of *Bletilla striata* polysaccharide modified with stearic acid (SA) and targeted with folate (FA-BSP-SA). The pH-responsive release effect of FA-BSP-SA micelles was observed, leading to increased release of Dox in acidic condition. The in vivo study conducted in mice showed a decrease of tumour weight and volume [77]. The new redox-sensitive polymeric micelles targeted with folic acid (FHSV—folic acid-hyaluronic acid SS-vitamin E succinate) for paclitaxel delivery (Ptx/FHSV) were designed by Yang et al. The nanoparticles characterize enhanced cell internalization caused by folic acid and redox-sensitivity leading to rapid drug release in presence of high concentration of glutathione (GSH). Ptx/FHSV micelles were compared to the single-targeted micelles and free paclitaxel. In vitro evaluation showed increased cellular uptake of the Ptx/FHSV micelles. In vivo study revealed enhanced tumour accumulation, inhibition of tumour growth and minimal toxicity to normal cells [89].

A novel approach was the development of FA-targeted filomicelles from a combination of poly(L-lactide)-Jeffamine-folic acid and poly(L-lactide)-poly(ethylene glycol) for delivery of betulin derivative, which reveals high cytotoxicity against cancer cells. Filomicelles (worm-like micelles) possess high drug loading capacity and long circulation time in the bloodstream. The successful in vitro internalization of PLA-Jeff-FA/PLAPEG micelles by FR-positive human cervix adenocarcinoma cells (HeLa) was confirmed by flow cytometry and confocal laser scanning microscopy (CLSM). Importantly, drug-free micelles did not affect the viability of cells (Figure 3) [81].

Fasehee et al. investigated disulfiram loaded NPs as a therapeutic system to treat breast cancer. Disulfiram is well known drug for alcoholism treatment with recently confirmed anticancer action by induction of reactive oxygen generation (ROS), which is responsible for activation of apoptosis. The folate-targeted PLGA-PEG NPs loaded with disulfiram have shown a significant decrease of breast cancer tumour growth rate in Balb/c mice. Additionally, no body weight loss or death was observed, chronic toxicity was lower and tumour growth inhibition was more significant [42]. Another example of using the not obvious drug for cancer treatment can be NPs loaded with orlistat, which is the FDA-approved anti-obesity drug with the ability to block the lipogenic activity of fatty acid synthase (FAS) present in 50% of cancer cells. Unfortunately, orlistat has poor bioavailability (≈1%). The prevention of fast degradation was achieved by drug loading to NPs synthesized by copolymerization of 2-hydroxyethylacrylate (HEA) and 2-ethylhexylacrylate (EHA) with FA. The nanoparticles were developed for the effective treatment of triple-negative breast cancer. The in vivo study showed 70% of volume reduction of MDA-MB-231 tumour xenografts in mice, suggesting that the anti-obesity drug can be considered as a novel strategy to treat highly challenging cancer without overexpression of progesterone and oestrogen receptors (HER) [43].

Worth mentioning is a novel nanoformulation composed of solid lipid nanoparticles (SLNs), obtained from lipid molecules which occur in the solid state at room temperature It is claimed that the advantage of SLNPs is their low biotoxicity and convenient large-scale production. In 2018 Rajpoot and Jain published results of their study of oxaliplatin loaded SLNs containing tristearin, 1,2-distearoyl-sn-glycero-3-phosphoethanolamine (DSPE), Lipoid S75 and Tween 80 conjugated with folic acid for colorectal cancer treatment. The formulation enabled to obtain higher anticancer activity on HT-29 (human colon cancer cell line) compared to free oxaliplatin and not-targeted oxaliplatin loaded SLNPs [90]. The further studies reported that the SLNs can be used for delivery of irinotecan to colorectal cancer. The SLNs improved in their sustained drug release properties compared to liposomes and niosomes, showing good stability and the possibility of conjugation. In vitro studies of irinotecan loaded SLNs targeted with FA (FA-SLNs)-exhibited prolonged drug release profile, high encapsulation efficiency and small particle size (varied from 201.88 ± 9.92 to 164.14 ± 5.57 nm) [83]. The exploration of SLNs is continued and the oral pH-responsive alginate microbeads loaded with irinotecan and targeted with folic acid (FA-SLNs) were developed for the treatment of colorectal cancer [91]. Furthermore, the FA-SLNs were covered with Eudragit S100 to achieve pH-responsive alginate microbeads oral delivery system, folic acid targeted which was used for irinotecan delivery. The system was evaluated in vitro for drug release in various pH and the findings proved drug release in an intestinal region only (pH > 7.0). In vivo research was conducted on Balb/c nude mice model bearing HT-29 tumour to observe targeting potential and organ biodistribution. The Eudragit coated, irinotecan loaded FA-SLNs showed the enhanced tumour growth inhibition in comparison to no-targeted Eudragit coated SLNs with irinotecan and free drug [91].

##### Dual-Drug Delivery

Apart from the simple liposome encapsulation by one active substance, the innovative, compound formulations, are being synthesized. Combination of more than one cytostatic drug in a single cycle of chemotherapy is well known strategy, which relies on the combining of different mechanisms of action of the used drugs that may provide better anticancer effects. Therefore, co-encapsulation of more than one drug—cisplatin (Cis) and paclitaxel in folic acid-modified liposomes revealed the greater chemotherapeutical response of FR-positive non-small lung cancer cells [48]. FR-targeted liposomes loaded with paclitaxel and imatinib have shown effectiveness in promoting cell death and suppressing vascular endothelial growth factor (VEGF) expression in folate-receptor-overexpressing cancer cell lines [92]. In addition, the cytotoxic activity of double loaded FA-modified liposomes with mitomycin C and doxorubicin was proved against prostate-specific membrane antigen (PSMA)-positive cancer cells [8]. Gazzano et al. designed folate-targeted liposomes with doxorubicin conjugated with nitric oxide that inhibited the Pgp efflux. In preclinical trial, this formulation showed superior efficiency to doxorubicin and Caelyx^®^, with similar toxicity, so it can be potentially advantageous for the treatment of FAR-positive/Pgp-positive breast tumours [93].

NPs were used to achieve an efficient drug delivery system for cisplatin and docetaxel in breast cancer treatment [47] or cisplatin and paclitaxel against non-small lung cancer [48,49]. Thapa et al. prepared folic acid-targeted liquid crystalline nanoparticles (LCN) loaded with docetaxel and cisplatin for effective metastatic breast cancer treatment. The LCN characterized small size (~250 nm), good encapsulation properties and controlled drug release. In vivo trial conducted on MDA-MB-231 tumour bearing xenograft mouse model confirmed that inhibition of tumour growth was more significant in mice treated simultaneously with cisplatin and docetaxel than in mice treated with separately administered drugs. However, even more significant tumour inhibition was obtained in mice treated with FA-targeted LCNs co-encapsulated with both drugs, indicating their therapeutic potential [47]. Cisplatin has also been co-delivered with paclitaxel for the treatment of lung cancer in a nanosystem composed of folic acid modified PEG-PLGA. The analysis of the proper drug ratio was evaluated toward four different lung cancer cell lines (L929, R1610, A549 and M109). It has been found that Cis/Ptx concentration of 1:2 shows the greatest cell growth inhibition. Additionally, the synergistic effects of those two drugs could promote and accelerate the tumour cells death, that was confirmed in vivo. The M109 and A549 lung cancer cell grafted tumour-bearing nude mice were treated with PBS, free cisplatin, free paclitaxel, FA-Cis-NPs, FA-Ptx-NPs, Cis-Ptx-NPs, FA-Cis-Ptx-NPs and combination of free drugs to compare anticancer activity and systemic toxicity of various formulations. It has been observed that co-delivering of two drugs in the targeted NPs (FA-Cis-Ptx-NPs) exhibited the highest antitumour efficiency with minimal side effects [48]. The research was continued to confirm hemocompatibility of these nanoparticles and no toxic effect (e.g., blood haemolysis, blood clotting or complement activation) [49].

#### 3.2.2. Gene Delivery

FA-targeted liposomes may be also used as carriers of genes, which are susceptible for degradation by several nucleases in the serum, so need protection and delivery systems providing enhanced cell uptake and controlled release. A promising strategy for improved anti-tumour effect was achieved by co-delivering of small interfering RNA with cisplatin, doxorubicin and ursolic acid in folate-targeted liposomes [94,95,96]. In addition, dendrimers made from cationic polymers can be considered as carriers appropriate for gene delivery, e.g., siRNA [97,98], because they can provide good protective properties against rapid enzyme degradation and effective gene transport to intracellular space. The problem of poor cationic polymer safety was overcome by the idea of a modification of terminal amines of the dendrimers with gold nanoparticles and conjugation of folic acid. In vitro study has shown that PAMAMs dendrimers modified with Au and FA were not cytotoxic (cell viability up to 90%) and induced transgene silencing up to 75% in HeLa (human adenocarcinoma cell line) [97].

#### 3.2.3. FA-Targeted NPs for Thermo-, Photo-, Radiotherapy and Diagnostic or Theranostic Application

There are also a number of a novel approach of polymer-coated magnetic nanoparticles (MNPs), which possess magnetic inner core (usually Fe_3_O_4_ or Fe_2_O_3_) covered by a polymeric shell (e.g., PEG, starch, dextran). MNPs can be targeted to the tumour cells and release a drug in response to environmental factors [63,64,65]. Combination of magnetic properties and targeting to folic acid receptors has been assessed. According to the in vitro research conducted by Gunduz et al., idarubicin-loaded FA-PEG-MNPs showed increased internalization by MCF-7 (human breast adenocarcinoma cell lines) cells located near to the magnet site and double increased cytotoxicity in comparison to the free idarubicin [63]. The influence of PEG-ylated MNPs on MCF-7 cells was also investigated by Saragazi et al. The findings confirmed that FA-conjugated MNPs loaded with methotrexate (MTX) had a significant inhibitory effect on MCF-7 cells and showed controlled enzyme-dependent release of MTX [82]. The in vitro and in vivo properties of 188Re labelled folate-targeted albumin nanoparticle coupled with cisplatin were analysed. These MNPs combine three strategies of cancer treatment: chemotherapy, radiotherapy and thermotherapy. Three groups of mice showed a significant reduction of tumour mass of more than 80% (I—treated with chemotherapy and thermotherapy; II—treated with radiotherapy and thermotherapy; III—treated with thermotherapy, chemotherapy and radiotherapy) and the triple therapy showed the most significant inhibition (88.52%). Furthermore, only a few mice exhibited weight loss and decreased appetite, but none of them died. These findings give a chance for the treatment of the difficult to cure ovarian cancer, overcoming MDR effect and increase of a chance for recovery [44].

Nanoscale metal-organic frameworks (NMOFs) are another promising drug delivery carriers. NMOFs are a class of porous and crystalline materials obtained from metal ions (clusters) and organic linkers. The advantages of NMOFs involve high area size for functionalization, large pore size for drug loading and biodegradability. Folic acid was successfully added to zirconium-based MOFs, MOF-808 and Nh2- Uio-66 followed by encapsulation of 5-FU. The NMOFs loaded with 5-FU exhibited pH-sensitive drug release, enhanced cellular uptake and cytotoxicity against HeLa cells [99].

The novel therapeutic idea was developed for a combination of cancer treatment and diagnosis [57,58,59,60,61]. Adequate diagnosis and precise imaging tools to localize tumour cells, lymph node checking and margin assessment are a very important part of cancer treatment. There are still serious limitations of cancer diagnosis by using contrast agents, such as problems with imaging of a whole tumour mass, with crossing brain blood barrier or small cancer detection. FA-targeted NPs are a promising tool to overcome those limitations. Intraoperative imaging was improved by Keating et al., who produced NIR FA-targeted contrast agent [57]. Folate-carbon dots (FA-CDs) made from poly-(acrylate sodium) (PAAS) were designed as a passivating agent and a turn-on fluorescence probe for detection of cancer cells [58]. Aconitic acid was used to prepare fluorescent carbon dots conjugated with FA, which showed potential as a turn-on fluorescent imaging tool for different kinds of tumour cells with FRs overexpression [60]. Perylenemonoimide (PMI) dye-doped polymer nanoparticle (PNP) with NIR emission for live-cell imaging was demonstrated by Pal et al. [59]. The positron emission tomography (PET) radiotracers can also be in the form of FA-targeted nanoparticles, e.g., folate-PEG-NOTA-Al18F [61].

The folate-targeted lipid-polymer hybrid nanoparticles (LPHNPs) loaded with indocyanine green (ICG) and perfluoropentane (PFP)-carrying oxygen (TOI_HNPs) were developed. The LPHNPs are core-shell structures with lipid shell and polymeric core, combining properties of liposomes and nanoparticles, which allow to overcome limitations of both types of drug carriers and enhance their delivery properties, e.g., controlled release, long circulation time, encapsulation efficiency. Additionally, the LPHNPs was modified with folic acid to target FR-overexpressing ovarian cancer cells. ICG is a sensitizer for phototherapy and perfluorocarbons (PFCs) are oxygen carriers. Studies confirmed the stability of LPHPNs, their active targeting ability (compared to PLGA NPs) and activation by laser exposure. In vitro trial on SKOV3 cells showed that TOI_HNPs can release oxygen. However, some unexpected disadvantages connected with photo-sonodynamic therapy (PSDT) were reported, e.g., increased risk of activating drug resistance pathway. Thus, future in vivo studies are required as well as some improvements of NPs, e.g., encapsulation of anticancer drug [100].

FA- targeted dendrimers can also be used as carriers of contrast agents [101,102,103] and in radiotherapy [104]. A new therapeutic nanocomplex based on dendrimers modified by FA, carrying two active chemotherapeutic agents—fluorouracil and ^99m^Tc to breast cancer cells has been achieved. In vivo studies in breast tumour-bearing BALB/C mice resulted in excellent tumour inhibition rate (reduced growth), significant reduction of tumour size and prolonged survival time. Furthermore, data obtained after testing with a gamma camera indicated that nanocomplex can be useful as an imaging tool [105,106].

The recent achievement was also gained by the development of methotrexate-loaded Au@SiO_2_ nanoparticles conjugated with folic acid for use in breast cancer phototherapy with low-level laser therapy (LLLT). The apoptosis was observed in MCF-7 and MDA-MB-231 cells treated with Au@SiO_2_ NPs, MTX-FA loaded Au@SiO_2_ NPs with and without laser therapy. The most significant cytotoxicity exhibited MTX and FA loaded Au@SiO_2_ NPs used in combination with LLLT. Synergistic effect of MTX-FA loaded Au@SiO_2_ and LLLT observed in both cell lines and decreased cell viability may be a rationale for future investigations of designing nanoparticles for cancers phototherapy with low-level lasers [54].

### 3.3. Clinical Trials and Patents

Some of the FA-targeted drugs have been the objects of clinical trials (Table 2). In the tested formulations, one or more active agents were conjugated with folic acid via spacers, which may be polysaccharides, proteins or PEGs, separating the drug from folic acid to avoid steric interference between them. Vintafolide (MK-8109, EC145) is a conjugate of vinblastine and folic acid, which was examined in platinum-resistant ovarian cancer treatment and reached Phase III of a clinical trial. In 2014, the trial was discontinued, due to no increase in tumour progression-free time. However, it has been found that patients who did not respond to treatment had a high P-glycoprotein level, which could be a reason for a failure [107]. The second generation of spacers were used to create another potentially useful conjugate, i.e., E0489 (folate–desacetylvinblastine hydrazide with modified linker), which exhibited 70% lower toxicity in preclinical studies compared to the EC145. The E0489 was tested in clinical trial NCT00852189 opened to patients with refractory or metastatic cancer who have exhausted standard therapeutic options [108]. Another example is a folate-indole-cyanine green-like conjugate (OTL38), which is an intra-operative imaging tool for FR-positive ovarian cancer. The Phase II of clinical trial allowed the detection of an additional lesion in 48.3% of patients with the use of OTL38 [109] and phase III (NCT03180307) was completed at the end of 2020. In addition, to single drug conjugates, the conjugate of folate-desacetylvinblastine hydrazide or folate-mitomycin C (E0225) was also tested in NCT00441870 trial. In this study, the E0225 was administrated with 99mTC-EC20 (folic acid-technetium 99m conjugate). The number of clinical trial of folic-acid conjugates developed for therapy of various types of cancer is increasing, as presented in Table 2.

In recent years, many different types of Fa-targeted drug transport systems have also been patented (Table 3). Some of the patents concern nanoparticles encapsulated with an anti-cancer drug or having magnetic properties that are used simultaneously for therapeutic and diagnostic purposes. A large number of patents confirm the great interest in nanoparticles targeting folic acid receptors and show the tendency to create more and more advanced transport systems in anti-cancer therapy combining various mechanisms of targeted therapy.

### 3.4. Summary

The common choice of folic acid as a targeting ligand is related to its outstanding properties, e.g., lack of toxicity or immune reactions, availability, facility to chemical modification and to scale-up for clinical applications. Another reason is the fact, that the FA receptors are overexpressed in human carcinomas including breast, ovary, endometrium, kidney, lung, head and neck, brain, colon and myeloid cancers while only minimally distributed in normal tissues. Various kinds of FA-targeted nanocarriers have been developed (Table 1), for single-drug delivery and co-delivery of other anticancer drug or gene. In addition, advanced NPs decorated with folic acid have been developed from smart materials that release a drug in response to environmental factors or enable combination of chemotherapy with thermo-, photo-, radiotherapy, diagnostic or theranostic application. The large numbers of patented and involved in clinical trials FA-targeted nanoparticles (Table 2 and Table 3) proves a significant progress in this field.

## 4. Biotin—Targeted Nanoparticles

### 4.1. Biotin as a Targeting Ligand

Biotin, also known as vitamin H or coenzyme R, is a basic co-factor for the activity of carboxylases. It is associated with metabolic processes such as gluconeogenesis, synthesis of the fatty acids or catabolism of branched amino acids. It also promotes cell growth and is delivered especially into cells with high proliferation rates including tumour cells [110]. Biotin can be conjugated to the different molecules via valeric acid tail to achieve biotinylation. The surface of drug delivery systems (DDSs) may be biotin-functionalized through biotin coupling to the polymer chain before obtaining particular nanocarriers (pre-conjugation) [111] or by connecting biotin onto the surface of nanocarriers after preparation (post-conjugation). The two biotinylation strategies of micelles are presented in Figure 4 [112].

Biotin enhances the internalization of nanoscale drug delivery systems by the target cells/tissue while exerting a lesser effect on normal cells and thus, became one of the most attractive targeting moiety. Since biotin receptors—sodium dependent multivitamin transporters (SMVT)—are overexpressed on the cancer cell surface, they, in turn, became a target of biotin-functionalized DDSs [113]. This fact has been utilized as a new strategy of cancer therapy, diagnostic and theranostic, that combines both, therapy and diagnostic [114]. Many reports have confirmed that biotinylated drug vehicles increase selectivity and uptake of active agents in tumour cells when compared to non-biotinylated DDSs [115,116]. Moreover, enhancement of the cellular uptake of various drug carriers results in active recognition of biotin by the receptors, regardless of the type of DDS modification, so biotin may be covalently linked with a carrier or surface-attached. In addition, in some cancer cells such as colon, breast, lung, renal or ovarian, expression of SMVT is higher than other transporters e.g., folate receptors (FARs). These findings made the biotinylation a strategy of aggressive cancer targeting, especially those with SMVT but without FAR overexpression [117].

### 4.2. Biotin-Targeted Nanoparticles

The anticancer properties of biotinylated nanosystems have received great attention from researchers (Table 4) [118]. The era of biotinylated DDS has been started from the article published in 2004 by Russell-Jones et al. It has been reported that the therapy of colon cancer (using Colo-26 xenograft model) with the biotin-labelled doxorubicin-hydroxypropylmethacrylic acid (Dox-HMPA) complex provides enhanced efficiency when compared to the control group. Furthermore, this effect was not observed when folic acid or vitamin B12 were applied as targeting moieties [119].

#### 4.2.1. Drug-Delivery Application

The biotin-mediated DDS for targeted tumour delivery of doxorubicin was obtained by a modified nanoprecipitation method combined with self-assembly [120]. The structure of the multilayer Dox-PLGA-lecithin-PEG-biotin nanoparticles with an average diameter of 110 nm is presented in Figure 5. Cytotoxicity of nanoparticles was studied in vitro in hepatoma cell cultures (HepG2—human liver hepatocellular carcinoma cell line) and in vivo in tumour-bearing mice. Both studies showed a greater inhibition effect on cancer cell proliferation than nanoparticles without biotin or free drug.

Quercetin belongs to flavonoids that are present in many vegetables and fruits. It has been reported that quercetin inhibits drug efflux by interacting with some protein of ATP-binding cassette (ABC) transporter, but also inhibits gene expression of P-gp and MDR1 and thus may serve as a chemosensitizer in the therapy of cancer showing MDR effect [134]. However, extremely hydrophobicity of quercetin seems to be the main limitation to start clinical trials. To overcome this drawback, polymer nanoparticles were used as a dual-drug delivery system. In order to enhance the anticancer property of doxorubicin and prevent from the MDR effect of cancer cells, Dox and quercetin have been incorporated into biotin-decorated methoxy poly(ethylene glycol)-b-poly(ε-caprolactone) (PEG/PCL) using thin-film hydration method [122]. Studies have shown an increase of doxorubicin concentration within the cells and improved retention which arose from higher drug uptake and lower efflux rate in the studied breast cancer cells (MCF-7/ADR). These results were consistent with the in vivo study demonstrating significantly reduced Dox resistance in MCF-7/ADR-bearing mice.

Paclitaxel (Ptx) is another common anti-neoplastic agent used for the treatment of various cancer types, such as breast, ovarian, lung, head cancers or AIDS-associated Kaposi sarcoma. Ptx acts as the microtubule-stabilizer and is considered as the most significant advance in the chemotherapy of the past years [135]. The first biotin-mediated DDS containing Ptx was reported by Kim et al. in 2007 [115]. In this study, micelles obtained from biotin-conjugated PEG/PCL block copolymer served as a drug carrier. Nanosystems with the size of 88–118 nm were tested in vitro to determine the cytotoxicity as well as cellular uptake. Biotin-conjugated PEG/PCL micelles exhibited relatively high cell viabilities, while Ptx-loaded biotinylated PEG/PCL carriers highly selective toxicity for HeLa 229 and MCF-7 cells.

Polymeric micelles based only on block copolymers, amphiphilic poly(N-2-hydroxypropyl methacrylamide)-block-poly(N-2-benzoyloxypropyl methacrylamide) (p(HPMAm)-b-p(HPMAm-Bz) were synthesized with biotin-CDTPA or CDTPA (4-cyano-4-[(dodecylsulfanylthiocarbonyl)-sulfanyl]pentanoic acid) [123]. In aqueous environment, the polymer self-assembled into micelles with the size of 40–90 nm, which was dependent on the length of hydrophobic chain in copolymers. Drug-free and paclitaxel-containing micelles of 10 wt% drug loading were obtained and examined in vitro. It was observed that biotin-tagged DDSs were internalized more efficiently than non-biotinylated ones by the cells overexpressing biotin receptors (A549 lung cancer cells), whereas both types of micelles characterized very low cellular uptake by HEK293 human embryonic kidney cells lacking SMVT. As a result, targeted micelles containing Ptx showed stronger cytotoxic activity against lung cancer cells than micelles without biotin.

In another study, biotinylated poly(amidoamine) (PAMAM) dendrimers of generation 4 (G4) were employed to targeted delivery of Ptx, which was covalently attached to the surface of dendrimer via succinic acid linker [124]. To prevent the systemic circulation of dendrimers but also to minimize their toxicity due to cationic properties, poly(ethylene glycol) was linked. In vitro studies revealed higher efficiency in cellular internalization as well as cytotoxicity of A549 cells referred to dendrimer-Ptx conjugated with biotin when compared to carriers without vitamin. Moreover, in 3D tumour cell spheroids, biotin-decorated dendrimers displayed better penetration, cytotoxicity and growth inhibition than non-targeted PAMAM and free drug.

Recently, dendrimers were also applied as DDS for gemcitabine [125]. This drug can replace cytidine in DNA thus suppress proliferation. It showed activity in various solid tumours and has been approved for therapy of many cancer types as pancreatic, bladder, breast, colon, ovarian and cervical cancer [136]. Gemcitabine was loaded into half-generation PAMAM dendrimer (PG4.5) modified with diethylenetriamine (DETA) served as a linker to biotin conjugation. The obtained nanoparticles were tested in HeLa cells cultures. The PG4.5-DETA-biotin was non-toxic while PG4.5-DETA-biotin/gemcitabine exhibited cytotoxicity and anti-proliferative activity based mainly on apoptosis induction. However, the cytotoxicity of drug free-PG4.5-DETA-biotin/gemcitabine was slightly lower than that of free drug, which may be the effect of lower molecular size and thus, faster cellular uptake of gemcitabine [125].

There are also studies concerning other active agents delivered via biotinylated, polymeric nanocarriers with in vitro and in vivo confirmed anti-cancer activity. Among them, artemisinin should be mentioned but also naringenin co-delivered with gefitinib to enhance the anti-tumour effect of gefitinib [126,127]. In these cases, biotin-conjugated PEG/PCL block copolymer was used as a drug carrier in form of micelles for artemisinin and nanoparticles for naringenin and gefitinib. The results of both works constitute the basis for the continuation of research in the next clinical phases.

Apart from polymers, there are also lipid-based carriers with biotin modification. Recently, biotin-polyethylene glycol 2000-distearyl phosphatidyl ethanolamine (biotin-PEG-DSPE) was used in the emulsification-ultrasonic and low temperature-solidification method to obtain nanostructured lipid carriers (NLCs) for disulfiram delivery in the presence of copper ion [128]. DDSs exhibited good stability and cytotoxicity toward breast cancer cells (4T1) in vitro and in vivo.

Multi-seed polymeric liposomes loaded with asulacrine (ASL-BIO-MPL) was prepared through encapsulating micelles as seeds in the aqueous phase of biotinylated polymeric liposomes using micelle gradient method [137]. The outer layer of such systems was modified with polymer-polypeptide, which is cleaved by matrix metalloproteinases-9 and attached with the tumour targeting agent. After reaching the target site, metalloproteinases-9 degraded cleavable peptides into short peptides causing the changes in liposomal membrane architecture. This resulted in the release of inner asulacrine, containing small micelles for deep intratumour distribution. In this study, a two-step method was used to scavenge the blood of ASL-BIO-MPL with the use of injected avidin employed to protect normal tissues from nanocarriers (Figure 6). The augment cell penetration and cytotoxicity of ASL-BIO-MPL in 3D tumour spheroids and tumour-bearing mice were confirmed [129]. In vivo safety experiments shown that targeted nanocarriers in the presence of avidin caused mild pathological changes in studied tissues such as heart, liver, spleen, lung and kidney. Nevertheless, the use of avidin may be considered controversial due to its origin, non-specific binding and possible immunogenicity [138].

Lu et al. designed and synthesized single [(Bio-Chol)Lip] and double [(Bio_2_-Chol)Lip] branched biotin-attached cholesterol to obtain liposomes differing in biotin density, as DDSs targeting breast cancer [139]. The in vitro and in vivo studies revealed that increasing the biotin density on the liposome surface significantly improved tumour targeting. The (Bio_2_-Chol)Lip exerted low systemic toxicity since normal cells showed very low uptake. Moreover, cytotoxicity and apoptosis assays exhibited that (Bio_2_-Chol)Lip containing paclitaxel, as a model anticancer drug, had better therapeutic properties than other prepared Ptx-loaded liposomes.

Another study of carbon-based drug delivery systems with biotin moiety was carried out by Gupta et al. [132]. The reduced-graphene oxide nanocarriers containing gallic acid were coated with biotin-decorated PEG- bis-(amine) and, as two-dimensional DDSs (BPBA@GA-rGONC), were subjected to evaluation of cytotoxicity and cellular uptake with the use of A549 (human lung carcinoma) cell culture. The in vitro studies confirmed better targetability to cancer cells and significantly decreased IC_50_ value of the obtained nanocarriers compared to free gallic acid as well as nanocarriers without coating (113.9 μg/mL versus 171.6 μg/mL and 137.5 μg/mL).

Gold nanoparticles are investigated as a drug delivery platform that may be decorated with different targeting agents as monoclonal antibodies, peptides, folic acid or biotin [140,141]. Such modification improves the anti-cancer activity of delivered agents, which was confirmed by the work of Pramanik et al. [133] The synthesized copper (II) complex was attached to 20 nm gold NPs and stabilized by amine terminated lipoic acid-PEG. The NPs were then biotinylated to achieve targeted delivery properties toward cancer cells. All of the obtained types of NPs, with and without biotin functionalization, were then examined in HeLa and HaCaT (human nontumourigenic immortalized keratinocyte) cells line cultures and mice. Biotin-decorated gold NPs highly suppressed tumour growth of HeLa cell xenografts in mice. In a tested group of animals, no significant weight loss was observed which suggests the non-toxic systematic effect of the biotin-conjugated gold NPs.

##### Biotin-Targeted NPs for Chemo-Photodynamic Combination Therapy

Biotin-conjugated and PEG-ylated porphyrin nanoparticles for mitochondria and lysosomes co-targeting loaded with doxorubicin were developed for chemo-photodynamic combination therapy [121]. In this study, *meso*-tetraphenylporphyrin (TPP) served as a photosensitizer to produce highly reactive oxygen species in light conditions, while doxorubicin was used as a chemo-agent. The acid–amine reaction of biotin–PEG–COOH with TPP-amine enabled the conjugation of TPP–PEG–biotin and the self-assembly of TPP–PEG–biotin with doxorubicin encapsulation at the level of 25.03%. Studies of the intracellular localization revealed that conjugate, self-assembled nanoparticles and NPs with Dox were distributed mainly to the mitochondria and partly to the nuclei and lysosomes of MCF-7 cells, while meso-tetra(4-sulfonatophenyl)porphyrin (TPPS) was found only in lysosomes. It was suggested that PEG-biotin modification of TPP helps not only in selective cellular, but also intracellular targeting. However, the cellular uptake of TPP–PEG–biotin NPs was slower than TPP–PEG–biotin conjugate. Nanoparticles containing doxorubicin generated cytosolic calcium and caspase 3 at a higher level in light conditions than in dark, which caused more apoptosis of cancer cells.

#### 4.2.2. Gene Delivery

Chitosan entered in biomedical fields in the 1990s and had been used in wound dressing as an antimicrobial agent [142] or tissue engineering as extracellular tissue matrixes [143]. It is also extensively investigated as a platform for delivery of drugs [144]. As chitosan is relatively less toxic than other cationic polymers, it is thought of as a promising excipient for gene delivery systems [145]. This natural polymer protects the naked genes from DNAses and thus improves the cellular uptake of DNA-based drugs administered to the body. To increase the cellular targeting of chitosan-based gene delivery systems to liver cancer, the biotinylation has been utilized by Cheng et al. [130]. The biotin-modified chitosan nanoparticles with plasmid DNA were prepared for stimulation of immune response in liver cancer cells. The synthesized plasmid (pGM-CSF-GFP-IRES-Rae-1-IL-21) contained genes of granulocyte-macrophage colony stimulating factor (GM-CSF) and interleukin-21 (IL-21) to trigger activation of cytotoxic T lymphocytes and natural killer cells. The obtained biotinylated chitosan NPs exhibited significantly improved gene and protein expression of GM-CSF, IL-1 and Rae-1 when compared to the nanocarriers without biotin moieties. Additionally, biotinylated nanocarriers highly increased the survival time of the tumour-bearing mouse. It was concluded that biotinylated chitosan NPs can mediate gene transfer and exert an inhibitory effect on the hepatoma cell model in situ, without any side effect on other cells.

### 4.3. Summary

Biotin promotes cell growth and is delivered especially into cells with high proliferation rates, including tumour cells. Biotin receptors—sodium dependent multivitamin transporters (SMVT)—are overexpressed on the surface cancer cells, e.g., colon, breast, lung, renal or ovarian and they are a target of biotin-functionalized DDSs. The diversity of biotin-targeted nano-delivery systems designed for single- and multi-drug delivery, gene delivery or chemo-photodynamic combination therapy is presented in Table 4.

## 5. Dual-Targeted Nanoparticles

### 5.1. Tumour Heterogeneity

Tumour heterogeneity, which occurs not only between patients, but even between primary tumour and metastases and within the tumour itself, is a critical aspect of cancer biology and remains a complex and challenging hurdle in the development of effective cancer therapy strategies [146,147]. Intratumoural and intertumoural heterogeneity (including cellular morphology, cell signalling, cell surface markers, receptors, metabolism, motility, drug resistance, angiogenic, proliferative, immunogenic and metastatic potential) is the result of genetic and epigenetic changes that occur both in cancer cells and tumour stromal cells [148,149]. In heterogenic tumours, a pool of heterogeneous cells exists where each clonal cell population will differ in the expression of various molecular targets, the expression levels (quantity) and quality of these molecules (accessibility and affinity). Thus, the relative levels of vitamin receptor overexpression may differ from cell to cell in the tumour. Since active targeting is based on the recognition and binding of ligands to tumour cell surface receptors, the targeting effect is affected by the receptor expression (surface markers), which may change dynamically with tumour progression [29]. Moreover, ligand-receptor binding is a saturable process as the recycling and synthesis of receptors takes time [6]. It was also reported that different receptors are often upregulated on tumour cells and drug resistance is often associated with upregulation of alternative receptors as well as pathway switching between two receptors [150]. These factors will affect the delivery efficiency of single-ligand nanomedicines, causing variation in response to targeted therapy within a tumour and reducing drug efficacy [23,147]. Therapy-sensitive cells will die upon the treatment; however, in light of the selective mode of therapy, a fraction of the cells can evade death and emerge as therapy-resistant cells [151]. These surviving cells generally harbour an aggressive phenotype and they may remain dormant or disseminate into the bloodstream and culminate in tumour metastasis, which severely complicates further treatment options [152,153]. Several methods, which generally rely on the cooperative work of nanosystems, are proposed as possible solutions; however, “tumour target amplification” appears to be a superior alternative. Tumour target amplification approaches can be classified into four categories: (1) self-amplifying systems that focus on increasing the levels of existing tumour-specific antigens (quantity); (2) artificial receptors that can be added to provide new targets (quantity); (3) peptide modification, where, instead of increasing the amount of cell-surface protein receptor targets, the endogenous receptors are manually engineered to increase binding affinity and recognition by the therapeutic ligand (quality); and (4) dual-targeting systems that characterize simultaneous targeting two cancer-specific factors (quality and quantity) [23]. The dual-targeting strategy will be discussed in Section 5.2.

### 5.2. Dual-Targeting

#### 5.2.1. Dual-Molecular Targeting

Based on the overexpression of specific receptors on tumour cells, active targeting nanomedicines have been developed with the ability to efficiently deliver active agents to the tumour cells via receptor-mediated endocytosis. Nevertheless, the efficacy of single-ligand nanoparticulate delivery systems is still limited due to the complexity of the tumour microenvironment and tumour heterogeneity. In recent years, dual-ligand nanomedicines have attracted a lot of interest due to presenting versatile functions and thus have the potential to improve the efficacy of tumour-targeted delivery [6]. Dual-targeting is still a novel approach in which a delivery system is equipped with two distinct ligands to target different receptors which may be either expressed on/in one type of cell or on different cells. This strategy aims to enhance targeted delivery of a cytotoxic drug cargo into tumour cells [154]. Combining two targeting ligands may improve the selectivity and uptake of the nanomedicine by specific tumour cells and provide the possibility to target different cells, which are involved in the development of the tumour or cells that possess two kinds of receptors on the surface. Combinations of ligands are classified into three different based on the types of targeted cells and the action sites (Figure 7): (1) two ligands target one kind of cell, which simultaneously overexpresses two kinds of receptors (Figure 7A), two ligands target two kinds of cells (Figure 7B) and combining cell membrane targeting with intracellular organelle targeting (nuclear targeting or mitochondrial targeting) (Figure 7C) [6].

So far, the most common dual-ligand combinations are those in which a second ligand is combined with either RGD, HA or transferrin (Tf), since they are overexpressed on various cancer cells and have been extensively studied [6]. There is also a growing interest in using combination with folate or biotin.

#### 5.2.2. Dual-Targeting with Folic Acid

The novel achievements in development of dual-targeted nanoparticles with folic acid are summarized in Table 5. Comparison of single-targeting (CD44 receptor) and dual-targeting (folate and CD44 receptors) micellar formulations obtained from hyaluronic acid-octadecyl (HA-C18) and loaded with paclitaxel showed that although all kinds of micelles possessed much longer half-life and moderately larger AUC than Taxol solution, the dual-targeted micelles provided better MDR-overcoming effect and exhibited excellent tumour-targeting ability. Thus, dual-targeting CD44 and FA receptors may be an effective strategy for intracellular drug-targeting delivery, overcoming drug resistance and tumour targeting [155].

Paclitaxel was also co-loaded with DNA in the hyaluronic acid (HA) and folate (FA)-modified polyethylenimine liposomes, to obtain the dual-targeting biomimetic nanovector. The dual-targeted liposomes could effectively target tumour cells, enhance transfection efficiency and subsequently achieve the co-delivery of Ptx and DNA, displaying great potential for optimal combination therapy [156]. Doxorubicin-loaded liposomes targeted with folate and transferrin were proven effective in penetrating the BBB and targeting the brain glioma. In vivo studies demonstrated that the FA and Tf-targeted liposomes could transport across the BBB and mainly accumulated in the brain glioma. The liposomes caused an increase of survival time and decrease of tumour volume [157]. Other liposomal nanocarriers loaded with doxorubicin bearing controlled numbers of both folic acid and a monoclonal antibody against the epidermal growth factor receptors (EGFR) were developed. Unlike single-ligand targeting, dual-ligand liposomes reduced viability only in target cells bearing both targeted receptors while sparing off-target cells. Selectivity enhancements determined by LC50 ratios for single- and dual-ligand formulations showed that dual-ligand liposomes were capable of achieving a 10-fold enhancement relative to off-target cells without the folate receptor and a 4-fold enhancement relative to off-target cells without the EGFR [158].

The nanoparticles targeted with folate and trastuzumab obtained from redox responsive multiblock copolymer (MB-PLA-ss-FA-Her-Dox-NPs) were developed. In vitro tests showed high drug encapsulation (≈22%) and significantly enhanced cellular uptake. Moreover, a 91% regression in Ehrlich ascites tumour was demonstrated and lack of significant heart, liver or kidney toxicity. Although the doxorubicin was chosen for the study, the obtained nanosystem can be employed to deliver also other kinds of drugs used in breast cancer therapy [165].

Novel folate (FA) and TAT peptide co-modified doxorubicin-loaded liposome (FA/TAT-LP-Dox) was developed [159]. The role of TAT peptide was to improve the capacity of translocating cell membranes and provide efficient intracellular delivery. Although the mechanisms for TAT peptide across cell membrane are still unclear, many studies have suggested that positive charges of TAT peptide play a key role in the uptake process. Liposomes with optimal ligand density (5% of FA and 2.5% of TAT) exhibited improved cytotoxicity and cellular uptake efficiency compared to single-ligand counterparts. Moreover, the targeting moieties, FA and TAT peptide, revealed synergistic effect in facilitating intracellular transport of the liposomes. The superiority of FA/TAT-LP in tumour targeting and accumulation was confirmed under in vivo conditions [159].

The liposomes modified with two kinds of ligands—folic acid and glutamic hexapeptide (Ptx-Glu_6_-FA-Lip) have been obtained for therapy of metastatic bone cancer [160]. It has been found that glutamic oligopeptide, especially glutamic hexapeptide, had an excellent bone-targeting ability, because multi-carboxy groups of peptides provide ionic interaction between negative charges and calcium ions in the mineral component (HAP) of bone [166]. The Ptx-Glu_6_-FA-Lip showed superior targeting ability in vitro and in vivo in comparison to free Ptx, non-coated, singly-modified and co-modified by physical blending liposomes [160].

A novel brain drug delivery system based on pluronic P105 polymeric micelles functionalized with glucose and folic acid for doxorubicin delivery (GF-Dox) were designed [162]. The glucose transporter (GLUT1), which is particularly highly concentrated in brain microvessels, is an important nutrient transporter in the human body, because glucose almost entirely supplies the high and continuous energy requirement of the brain and glucose can effectively penetrate through the BBB via facilitative GLUT1. Thus, the glucose-targeted ligand could potentially be used to facilitate the passage of carriers across the BBB. An in vivo study in rats showed a significant increase of Dox in the brain after micelles’ administration. In addition, bioavailability of Dox in GF-Dox micelles significantly increased (4.6-fold) in comparison to control Dox solution. The survival time of tumour-bearing mice of the GF-Dox group (32 days) was significantly longer than that of the free Dox group (19 days), or other control groups due to the dual-targeting effect of GF-Dox [162].

Folic acid-pectin-eight-arm polyethylene glycol-dihydroartemisinin/hydroxycamptothecin nanoparticles (FPPDH NPs) have been developed for targeted delivery of dihydroartemisinin (DHA). Folic acid and pectin were used as targeting ligands by taking advantage of the high expression of asialoglycoprotein receptors on the surface of liver binding pectin with galactose residues and high expression of folic acid receptors. FPPDH NPs had higher cytotoxicity than free DHA (204.5-fold in the case of H22 (mouse hepatocellular carcinoma cell line) and 178.4-fold in the case of HepG2) [163].

Fluorescent Au nanocomposite with Dox dual-targeted with folic acid and G-quadruplex oligonucleotide AS1411 (AF-D-AuNPs) for bioimaging was developed [161]. AS1411 is a novel nucleolin-targeted DNA aptamer, formed from a single-stranded, G-rich, phosphodiester, 26-mer oligonucleotide. It targets nucleolin, a multifunctional protein located primarily in the nucleolus, but also found in the cytoplasm and cell membrane, which is overexpressed in many types of cancer. AS1411entered a phase II clinical trial in metastatic renal cell carcinoma [167]. The authors observed very strong fluorescence signal of the AF-D-AuNPs incubated with cells. The nanocomposite may have great potential in early detection of cancer and bioanalysis field [161].

Gold nanoclusters (AuNCs) functionalized with folic acid and trastuzumab (Herceptin^®^) as dual-targeted radiosensitizer agents have been analysed [164]. Herceptin (HER) is widely applied in some types of cancer treatments as a chemotherapy agent but can also be used as a bioligand to increase tumour cell internalization of nanoparticles in HER2-positive breast cancer cells [168,169]. In addition, trastuzumab by enhancing radiation-induced apoptosis can increase the synergy between chemotherapy and radiotherapy as a chemo-radiotherapy modality. The dual-targeting strategy led to an enhancement accumulation of the nanoclusters in the cancer cells via active targeting mechanisms and to enhance significantly radiation therapy efficiency with the sensitization enhancement factor (SER) 1.77 and 1.5 fold larger than those obtained using non-targeted AuNCs [164].

#### 5.2.3. Dual-Targeting with Biotin

The recent studies on nanoparticles dual-targeted with biotin are presented in Table 6. Liposomes dual-targeted with biotin and glucose (Bio-Glu-Lip) and loaded with paclitaxel were evaluated for breast tumour-specific drug delivery, improvement of the efficacy and reduction of the chemotherapy side effects [85].

The glucose transporter 1 (GLUT1) is known to be overexpressed in various types of cancer cells due to the Warburg effect, an insufficient glycolysis pathway to generate adenosine triphosphate making glucose a suitable targeting ligand for drug delivery. Bio-Glu-Lip was recognized by the biotin transporter SMVT and the glucose transporter GLUT1 on the cell membrane via the residues on the liposome surface and was energy-dependently internalized via a synthetic endocytic pathway, including clathrin-mediated, caveolae-mediated and micropinocytosis-mediated endocytosis. Bio-Glu-Lip had the highest cell uptake in 4T1 and MCF-7 cells when compared to the non-targeting liposome (Lip), Bio-Lip and Glu-Lip. In addition, significantly increased accumulation of the Bio- and Glu-targeted liposomes in the breast tumour sites was observed [85].

A new strategy was developed to simultaneously introduce a nuclear protein—high-motility group box (HMGB)-1 for nuclear transport and biotin for particular tumour cell targeting [170]. The (HMGB)-1 is the focus of recent cancer research, because it plays a critical role in cancer development, progression and metastasis by activation of cancer cells, enhancement of tumour angiogenesis and suppression of host anti-cancer immunity [172]. The in vitro study showed that the presence of HMGB1 facilitates the nuclear transport of DNA, leading to enhanced transfection efficiency. In addition, the complexes exhibited an enhanced cellular uptake into HeLa cells due to the specific interactions between biotin moieties and biotin receptors on HeLa cells [170].

Chitosan nanoparticles (Bio-GC) modified with galactose and biotin for efficient targeting of fluorouracil to hepatoma cells were obtained. The specific binding of galactose ligand with asialoglycoprotein receptor (ASGPR) on hepatocyte membranes has been shown to induce liver-targeted drug transfer. The ASGPR is found on sinusoidal surfaces of mammalian liver cells and is a glycoprotein that specifically recognizes terminal galactose residues or acetylamino galactose. Each hepatocyte contains about 200,000 binding sites for ASGPR. In addition, the biotin has a great potential of increasing NP efficiency, because the expression of biotin receptor is 39.6 times higher in hepatocellular carcinoma cells than in normal liver cells. The Bio-GC nanoparticles with 5-FU had stronger in vitro and in vivo inhibitory effect on the proliferation and migration of liver cancer cells compared with 5-FU [171].

#### 5.2.4. Dual-Targeting with Combination of Folic Acid and Biotin

There is a concept of using combination of folic acid and biotin as targeting ligands [173]: one of the first papers dealing with the evaluation of the effectiveness of folate, vitamin B12 or biotin-functionalized polymeric materials as active drug targeting agents to tumour cells was published in 2004 by Russell-Jones et al. It has been reported that the cells overexpressing the receptors for folate or vitamin B12, overexpress also receptors for biotin [119]. The examples of cell lines with overexpression of either biotin receptor, folate receptor or both are presented in Table 7 and the cells negative for biotin and/or folate receptors expression are listed in Table 8.

The detailed analysis of the interaction of cells with surfaces modified with the folic acid and biotin was studied by Subedi et al. The mixed monolayers were prepared with a small amount (1%) of folic acid or biotin on a long poly(ethylene glycol) linker of Mw = 3400 Da and the remaining 99% was covered by a short oligo(ethylene glycol) (Mw ≈ 550–750 Da). This approach allowed to assess the targeting effect independently from endocytosis that typically accompanies a similar analysis for targeted nanoparticles. Significant targeting with greater attachment of human cervical cancer cells (HeLa) and human breast adenocarcinoma MCF7 cells was observed in comparison to the non-tumourigenic breast epithelial cells (MCF10A). Thus, the results confirmed that the targeting moieties can be used in drug delivery systems for targeting cancerous cells while sparing the surrounding noncancerous tissue. In addition, a drastically different behaviour was observed for competition with free vitamins, because the addition of free folic acid caused inhibition of cell attachment, but free biotin induced enhancement of cell attachment (anti-inhibition effect). The competition effect was observed also at low temperature (4 °C), which suggests that the proteins responsible for this effect are not recruited from cytosol during cell attachment [175].

An interesting aspect of development of dual-targeted drug delivery remains optimal ligand density on the surface of carriers for a maximal internalization. For a sake of increasing of nanoparticles functionality, it is necessary to clarify the effect of multiple ligands with different densities and ratios on the cell internalization efficiency. An attempt of solving this problem was undertaken by Liu et al. [28] with the use of fibre rods with hierarchically targeting capabilities. fibre rods obtained from poly(ethylene glycol)-poly(DL-lactide) or styrene-maleic anhydride copolymer were conjugated with folate/biotin ligands via PEG linkers and poly(sulfobetaine methacrylate) (PSBMA) ligands via acid-labile linkers. The zwitterionic polymers, containing both anionic and cationic charges in the same unit, have shown strong resistance to protein adsorption and low immunogenicity, so conjugation of PSBMA on fibre rods aimed to prolong blood circulation by preventing from protein opsonization and shielding the targeting ligands. The acid-responsive removal of zwitterionic ligands leads to exposure of targeting ligands (folic acid and biotin) and activation of tumour cell internalization. In this study, the densities of folate (0.09–0.66 μmol/g) and biotin (0.40–1.7 μmol/g) on the rods’ surface were analysed. It has been determined that the cellular uptake of FA-grafted fibre rods (FA-R) was time-dependent and increased with the incubation time. The highest uptake by 4T1 cells was observed for FA-R with the folate density of 0.48 μmol/g (up to 3.9 folds higher than other FA-R). The cellular uptake of biotin-grafted fibre rods (BIO-R) increased with increasing the biotin density to 0.89 μmol/g, but it was significantly reduced beyond this value. For the fibre rods grafted with both ligands, folate and biotin, the tumour cell uptake is maximized at the folate density of 0.36 μmol/g and biotin of 0.67 μmol/g. This suggested that the dual ligands with a critical density and an optimal ratio were essential for tumour cell internalization. The uptake of non-targeted rods was mediated via micropinocytosis, while the internalization of rods targeted with FA and BIO proceeded via clathrin-mediated endocytosis. It has been also exhibited that treatment with Dox-loaded rods grafted with FA, BIO and PSBMA enhanced the tumour growth inhibition, prolonged the animal survival and caused fewer lung metastases in comparison to the free Dox, non-targeted rods and rods grafted with FA and BIO [28].

##### NPs Targeted with Folic Acid and Biotin

Table 9 presents examples of the nanoparticles dual-targeted with folic acid and biotin. The multifunctional pH-responsive silica-coated nanoparticles with both, fluorescent and magnetic properties, triple conjugated to biotin, folic acid and doxorubicin (Fe_3_O_4_@SiO_2_(FITC)-BTN/folic acid/Dox) were synthesized for increasing tumour drug accumulation by active targeting and endosomal drug release properties. The Dox was conjugated with pH-labile Schiff-base formation, which caused stability of this acid-sensitive linkage at pH 7.4 (mimicking the physiological pH in the blood circulation) and breaking the bond at pH 5.0 (mimicking endosomal environment), leading to the significant drug release. The developed nanoparticles improved the accumulation of anticancer drug at the target site due to dual-targeting properties and ability to control drug release after cell internalization [197].

Dopamine-capped iron oxide nanoparticles containing two surface-grafted biologically relevant ligands, folic acid (FA) and biotin (BIO) (FA-Fe_3_O_4_-BIO) have been developed. The NP conjugated with FA and biotin NPs may interact with multiple receptors overexpressed on the surface of a diseased cell and offer enhanced cellular uptake via receptor-mediated endocytosis. The FA-Fe_3_O_4_-BIO were delivered into E-G7 and human HeLa cancer cell lines and tested toward their cellular uptake by immunofluorescence and flow cytometry analysis. Cell internalization of the FA-Fe_3_O_4_-BIO was time-dependent and the highest uptake was found after 24 h. The nanoparticles possessing single ligand on the surface, either FA or BIO showed several-fold lower uptake in the tested cell lines in comparison to the dual-conjugated FA-Fe_3_O_4_-BIO nanovectors. Importantly, the surface-functionalized magnetic nanoparticles did not exhibit cytotoxicity, which was demonstrated by high cell viability (>95%) [198].

Biodegradable dual-targeting micelles from combination of poly(L-lactide) co-poly(ethylene glycol)-folic acid (PLA-PEG-FA) and poly(L-lactide)-co-poly(ethylene glycol)-biotin (PLA-PEG-BIO) were developed for delivery of paclitaxel. The micelles showed high paclitaxel loading and low CMC value (0.001 mg/mL), which ensures their stability. The paclitaxel-loaded micelles characterized double morphology—filomicelles of over 100 nm length and 20–30 nm diameter and spherical micelles of ≈20 nm diameter. The in vitro cytotoxicity of paclitaxel-loaded PLA-PEG-FA+PLA-PEG-BIO micelles against ovarian cancer cells (OVCAR3) that characterize overexpression of both, folate and biotin receptors was confirmed [199].

Triple-targeted nanomicelles (162.7 ± 5 nm) for therapy of breast cancer were obtained from oligomeric hyaluronic acid (oHA), which is a macromolecular polysaccharide with good tumour targeting, biodegradability, non-immunogenicity and nontoxicity (Figure 8) were developed. Moreover, hyaluronic acid and its derivatives can also bind to specific receptors on external of cancer cells, owing to their high expression, for instance, CD44 receptors. The CD44 is a specific marker on breast cancer stem cells (BCSCs) that have the ability to self-renew and unlimitedly proliferate, which is the main reason for tumourigenesis, metastasis and relapse. The additional targeting properties were obtained by using two other targeting moieties—biotin and folic acid. The micelles were developed for delivery of two active agents—icariin (Ica) and curcumin (Cur) [200]. Ica is one of the main active ingredient of *Epimedium*, a traditional Chinese herbal medicine and it presents an antitumour effect by inhibition of proliferation and differentiation of tumour cells, promotion of tumour suppressor gene expression, inducing tumour cell cycle arrest [201]. Curcumin is another natural agent of natural origin that has potential in preventing and treating various by inhibiting tumour-associated gene expression and angiogenesis [200]. The pH-sensitivity of the nanomicelles were obtained by introduction of the hydrazone (Hyd) bond. In fact, the in vitro study revealed higher release of Ica and Cur from the Bio-oHA-Hyd-FA micelles in the acidic environment. The Ica and Cur-loaded Bio-oHA-Hyd-FA micelles presented higher cytotoxicity to cancer cells compared to the control groups (free Cur, free Ica, free Ica + Cur, Cur-loaded micelles and Ica-loaded micelles). The inhibitory effect on tumours was confirmed in vivo [200].

Self-assembled folate-biotin-pullulan (FBP) nanoparticles (NPs) have been developed for delivery of doxorubicin. Pullulan is a linear polysaccharide consisting of consecutive maltotriose units, which are connected by an α-1,6-glycosidic bond. Due to its outstanding biological properties, such as biocompatibility, biodegradability, low immunogenicity, nontoxicity and water solubility, pullulan has been widely used in the pharmaceutical industry. However, in this case, the biotin was used not as a targeting moiety, but rather as a hydrophobic moiety to form self-assembled NPs. When biotin is conjugated with other biomolecules via ester or amide linkages, its water solubility dramatically decreases because of the loss of hydrophilic carboxyl group [201].

### 5.3. Summary

Dual-targeted nanocarriers have been developed as one of the solutions that may overcome tumour heterogeneity, which occurs between patients, between primary tumour and metastases and within the tumour itself. As presented in Table 5, there is an increasing numbers of dual targeted nanocarriers with FA in combination with HA, Tf, glucose, etc., or NPs targeted with biotin with glucose, galactose or HMGB1 (Table 6). A novel approach is also combination of these two ligands in the same kind of nanocarrier (Table 9). There is also increasing number of NPs decorated with both, folic acid and biotin (Table 9). Overexpression of both kinds of receptors, FAR and SMVT, has been identified in many types of cancer cells (Table 7).

## 6. Single-Targeted versus Dual-Targeted Nanoparticles 

The progress in development of nanocarriers for anticancer drug delivery is presented in Figure 9.

The concept that nanocarriers can enhance the in vivo stability of anticancer compounds by protecting them from biodegradation or excretion, reducing their toxicity and enhancing the maximum tolerated dose by changing their systemic distribution, thereby improving the efficacy of anticancer compounds, is well known and has also been demonstrated clinically. The first generation of nanoparticles that are passively distributed to the tumour tissue by EPR effect is advantageous compared to the conventional dosage forms. However, more and more studies have revealed drawbacks of the enhanced permeability and retention (EPR), the most often proposed mechanism for nanomedicine delivery, which is mainly caused by tumour heterogeneity [21]. The current effort focuses on better understanding the tumour microenvironment and heterogeneity, because this knowledge is necessary to establish systems and strategies that characterize enhanced targetability. The currently, developed nanoparticles are focused mainly on active targeting of nanocarriers based on ligand-receptor recognition, which may show better efficacy than passive targeting in human cancer therapy. Moreover, the further progress may be obtained using dual-targeted nanoparticles and this concept has been supported by a solid experimental data. This review clearly presents that the dual-targeted nanocarriers are more effective compared to free drug, unmodified NPs and nanoparticles decorated with one kind of ligand. These NPs are superior in several aspects, involving cellular uptake, toxicity against tumour cells and decreased toxicity against normal cells. However, the dual-targeted nanoparticles are usually compared to the nanocarriers of the same type, which possess only one targeting ligand on the cell surface instead of the two. It should be emphasized that a great deal of effort is also being undertaken to improve the targetability and specificity of the single-targeted NPs. This direction involves using smart materials to augment functionality of NPs, e.g., pH- and redox-sensitivity. Additionally, there is also a dynamically increasing group of novel single-targeted nanocarriers developed for combined chemotherapy and photo-, thermo-, radiotherapy or for theranostic application. These “next generation” single-targeted NPs (advanced single-targeted NPs) and dual-targeted nanoparticles show superior efficiency in anticancer drug delivery than conventional therapy and single-targeted NPs.

## 7. Conclusions and Future Perspectives

Based on the studies conducted to date on the drug delivery systems of anticancer drugs, it has been recommended that future nanomedicine should be focused mainly on active targeting based on ligand-receptor recognition, because it is expected to show better efficacy than passive targeting in human cancer therapy. Some of the low-molecular-weight vitamins that play essential roles in cell survival and bind to the respective receptors with high affinity are folic acid and biotin. They are commonly used as targeting ligands for cancer chemotherapy, because of their selectivity: the specific receptors are overexpressed in a number of human cancer cells, but they are minimally distributed in normal tissues. The other advantages of these molecules include their availability, lack of toxicity, non-immunogenicity and ease of modification.

However, the nanoparticle design plays a significant role in tumour targeting, because of intra- and intertumoural variability present in the tumour cells and the tumour microenvironment that results in the heterogeneity of molecular, pathologic and clinical features of each tumour type. The recent achievements in targeted nanoparticle drug delivery indicate a great progress in this field. The nanoparticles of various morphology have been developed: liposomes, micelles, nanospheres, dendrimers, carbon nanotubes, nanorods, core-shell quantum dots and mesoporous nanoparticles.

There are also different strategies to achieve targeting effect. On the one hand, the nanoparticles having more than one targeting ligand are developed and these systems present increased efficiency confirmed by in vitro and in vivo study. In this group, the nanoparticles decorated with both targeting moieties, folic acid and biotin, are still a novel approach, although gaining an increasing interest. In addition, the studies on single-targeted NPs are also continued. The advanced systems use smart materials for achieving an additional properties, e.g., pH- or redox-sensitivity. There are also increasing numbers of systems combining cancer treatment and diagnosis. These advanced single-targeted NPs, with an additional functionality, similarly to dual-targeted nanocarriers, present superior properties over conventional drugs, non-targeted systems and single-targeted carriers.

Taking into account the promising results of both advanced single-targeted NPs and dual-targeted nanoparticles for anticancer drug delivery, further progress is expected in the nearer future.

However, apart from gaining new knowledge about the advanced targeted nanocarriers, additional efforts should be focused on their successful transition into clinics. Despite the significant therapeutic advantages of the nanoparticles, their clinical translation is still limited and does not progress as rapidly as expected, considering the positive preclinical results. From this point of view, several experimental challenges need to be addressed. First, of all, it is necessary to better understand the in vivo fate and interactions of nanoparticles with tumour tissue, cells and blood. The recent achievements concern aspects related to the design and preparation of delivery system, e.g., optimal ligand density on the surface of carriers for a maximal cell internalization. This direction of the research is going to be continued because of the inter- and intratumoral differences, which cause that even the same kind of NPs may differ in cellular uptake. Moreover, differences between nanocarriers may affect their biodistribution and cellular uptake that may require individual approach. Moreover, design and development of targeted NPs should consider their safety, biocompatibility and stability upon storage and, after in vivo administration reproducibly and the possibility of large-scale manufacturing. Last but not least, the promising in vitro results should be confirmed in vivo using appropriate animal models.

## Figures and Tables

**Figure 1:** Chemical structure of folic acid and biotin.

**Figure 2:** Scheme of different kinds of FA-targeted nanoparticles. After modification from (reproduced from Farran et al. [13]).

**Figure 3:** Confocal images showing the subcellular distribution of PLA-Jeff-FA/PLA_3000_PEG_2000_ micelles with fluorescein after 24 h incubation with HeLa cells (**A**) and normal human connective tissue cells (**B**) (reproduced from Jelonek et al. [81]).

**Figure 4:** Schematic presentation of the two biotinylation strategies. With permission from [112].

**Figure 5:** A schematic presentation (**A**) and TEM image at a scale = 100 nm (**B**) of DOX-PLGA-lecithin-PEG-biotin nanoparticles (**B**). With permission from Dai et al. [120].

**Figure 6:** The structure of biotinylated multi-seed polymeric liposomes and mechanism of stimuli-responsive size/ligand adapting strategy with the two-step method of the biotin-avidin system. 1-targeting delivery of nanocarriers to the tumour; 2-off-targeting scavenging of nanocarriers in blood and normal tissues by avidin. With permission from Jin et al. [129].

**Figure 7:** Scheme of three types of dual-molecular targeting: (**A**) dual-targeting nanocarriers target one kind of cell; (**B**) dual-targeting nanocarriers target simultaneously various cells; (**C**) Dual-targeting nanocarriers target cells that overexpress one kind of receptor on the cell and another kind of receptor inside cells on nuclei or mitochondria. With permission from Zhu et al. [6].

**Figure 8:** Scheme of the concept of cell uptake and drug release from Bio-oHA-Hyd-FA carriers. With permission from Tomeh et al. [200].

**Figure 9:** Evolution of nanoparticulate delivery system of anticancer drugs toward improvement of efficiency and decrease of toxicity.

**Table 1:** The examples of various FA-targeted nanoparticles for anticancer therapy.

DDS	Material	Drug	Tumour	Status	Ref.
Liposomes	FA-PEG-DSPE Cholesterol DPPC	5-FU	Colon	In vitro—T-29 cells, Caco-2 human colorectal adenocarcinoma cell line, CT26 mouse colon carcinoma cell line, HeLa cells, MCF-7 cells	[67]
				In vivo—mice	
Liposomes	HSPC/Chol/mPEG 2000-DSPE/folate-PEG-CHEMS	Dnr	Leukaemia	In vitro—L1210JF murine lymphocytic leukaemia cells In vivo—mice	[68]
Liposomes	FA-PEG2000	Cis	Liver	In vitro—PLC/PRF/5 Alexander hepatoma cells	[69]
	Phosphatidylcholine, Cholesterol				
Liposomes	FA-PEG-DSPE	Blm	Unspecified	In vitro—HeLa cells, MCF-7 cells	[70]
	cholesterol				
Liposomes	FA-PEG-DSPE	Cur	Unspecified	In vitro—HeLa cells	[71]
	Cholesterol				
	SPC			In vivo—mice	
Liposomes	FA-PEG-DSPE	Iht	Solid	In vivo—mice	[72]
Dendrimers	AU-FA-PPI	Dox	In vitro	[73]
Dendrimers	FA-PPI	Mtx	Breast	In vitro—MCF-7 cells	[74]
				In vivo—rats	
Dendrimers	FA-PAMAM	Dox	Unspecified	In vitro—KB cells	[75]
Dendrimers	FA-PAMAM +	Gem	Unspecified	In vitro—A431 epidermoid carcinoma cell line	[76]
	Magnetic mesoporous silica coated graphene oxide				
Micelles	FA-BSP-SA	Dox	Unspecified	In vitro—4T1 cells, HepG2 cells	[77]
				In vivo–rats and mice	
Micelles	MPEG-PHIS	Ptx	Breast	In vitro—MCF-7 cells	[19]
	FA-PEG-VE				
				In vivo—mice	
Micelles	FA-PF127-CHOL	Dtx	Melanoma	In vitro—B16-F10 cells, HepG2 cells, L929 mouse fibroblasts cells	[78]
				In vivo—mice	
Micelles	FA-PCL-b-P(HEMA-co-DMAEMA	Dox	Unspecified	In vitro—HeLa cells	[79]
Micelles	FA-MPEG-b-P(LA-co-DHP);	Ptx	oesophageal	In vitro—EC9706 human oesophageal cancer cell line, MCF-7 cells	[80]
	MPEG-b-P(LA-co-MCC)				
				In vivo—mice	
Micelles	PLA-Jeff-FA/PLA_3000_PEG_2000_	Bet	Unspecified	In vitro–HeLa cells	[81]
Nanoparticles	FA–PEG–MNP	Idr	Breast	In vitro—MCF-7 cells	[63]
Nanoparticles	Fe_3_O_4_-DPA-PEG-	Mtx	Unspecified	In vitro—MCF-7 cells, A549 cells	[82]
Nanoparticles	PLGA-1,3-diaminopropane-FA	5-FU	Colon	In vitro—HT-29 cells	[45]
Nanoparticles	FA-TCS	Dtx	Breast	In vitro—MDA-MBB-231 breast cancer cell line	[46]
				Ex vivo—rats	
				In vivo—rabbits	
Solid lipid nanoparticles	DSPE-FA	Iht	Colon	In vitro—HT-29 cells	[83]
Lipid-polymer hybrid nanoparticles	PGLA, PEG, SA, FA	Vcr	Lymphoma	In vitro–Raji human Burkitt’s lymphoma cell line, Raji/Vcr cells, A20 mouse reticulum sarcoma cells, HUVEC human umbilical vein endothelial cells	[84]
				In vivo mice	

PLGA—poly(lactide-co-glycolide); PEG–poly(ethylene glycol); DSPE—distearoylphosphatidylethanolamine 1,2-Distearoyl-sn-Glycero-3-Phosphoethanolamine; DPPC—dipalmitoylphosphatidylcholine; SPC—soybean phosphatidylcholine; SA- stearic acid; FOLATE-PEG-CHEMS—folate polyethylene glycol-cholesterol hemisuccinat; PPI—poly(propylene imine); PAMAM—poly(amidoamine); BSP—Bletilla striata polysaccharide; MPEG-PHIS-poly(ethylene glycol) methyl ether-poly(histidine); FA-PEG-VE- folic acid-poly(ethylene glycol)-(+)-α-tocopherol; PF127-Chol-Synperonic PE/F 127-cholesteryl hemisuccinate; FA-PCL-b-P(HEMA-co-DMAEMA))—folate-poly(ε-caprolactone)-block-poly(2-hydroxyethylmethacrylate)-co-poly(2-(dimethylamino)-ethylmethacrylate; MPEG-b-P(LA-co-DHP)-; MPEG-b-P(LA-co-MCC- poly(ethylene glycol)-block-poly(L-lactide-co-2-methyl-2-carboxyl-propylene carbonate); PLA-Jeff-FA/PLA_3000_PEG_2000_—poly(L-lactide)-Jeffamine-folic acid and poly(L-lactide)-poly(ethylene glycol); MNP–magnetic nanoparticles; FA-DPA-PEG—dopamine-polyethylene glycol-folic acid; TCS—thiol-decorated chitosan 5-FU–5-fluorouracil; Dnr–daunorubicin; Cis–cisplatin; Blm–bleomycin; Cur – curcumin; Vcr–vincristin, Iht–irinotecan hydrochloride trihydrate, Dox-doxorubicin; Gem–gemcitabine, Mtx–methotrexate; Ptx–paclitaxel; Dtx–docetaxel; Idr–idarubicin; Bet–phosphate betulin derivative; AU–gold.

**Table 2:** List of clinical trials involving folic acid conjugates.

Number	Study Title	Cancer	Drug	Phase	Status
NCT00308269	Study of Vintafolide (MK-8109, EC145) for the Treatment of Recurrent or Refractory Solid Tumors (MK-8109-006, EC-FV-01)	Unspecified	EC145	I	Completed in 2007
NCT00852189	Study of EC0489 for the Treatment of Refractory or Metastatic Tumors	Unspecified	EC0489, EC20	I	Completed in 2012
NCT00441870	Study of EC0225 for the Treatment of Refractory or Metastatic Tumors	Unspecified	EC0225, EC20	I	Completed in 2012
NCT01689727	Safety and Efficacy of FolateScan (Technetium Tc 99m EC20) in Subjects With Pituitary Tumors	Pituitary Tumors	EC20	II	Completed in 2012
NCT01689636	Safety and Biodistribution of Technetium Tc 99m EC20 in Normal Volunteers and Ovarian Cancer Patients	Ovarian Cancer	EC20	I	Completed in 2012
		Healthy Volunteers			
NCT01686256	Safety and Efficacy of FolateScan (Technetium Tc 99m EC20) in Women With Suspected Ovarian or Endometrial Cancer	Ovarian Cancer	EC20	I	Completed in 2012
		Endometrial Cancer			
NCT01689662	Safety and Efficacy of FolateScan (Technetium Tc 99m EC20) in Subjects With Suspected Metastatic Renal Cell Carcinoma	Metastatic Renal Cell Carcinoma	EC20	II	Completed in 2012
NCT01689714	Safety and Efficacy of Folatescan (Technetium TC 99M EC20) in Patients With Suspected Ovarian Carcinoma or Recurrent Endometrial Carcinoma	Ovarian Carcinoma	EC20	II	Completed in 2012
		Recurrent Endometrial Carcinoma			
NCT00485563	A Phase II Study of EC17 (Folate-hapten Conjugate) in Patients With Progressive Metastatic Renal Cell Carcinoma	Renal Cell Carcinoma	EC17	II	Terminated in 2012
			Biological: EC90 (KLH-FITC)		
			Biological: GPI-0100; Interleukin-2 Interferon-alpha		
NCT01002924	Extension Study of EC145 (Vintafolide) for Subjects Enrolled in a Previous Study With EC145 (MK-8109-010)	Solid Tumors	EC145	II	Completed in 2013
NCT02049281	A Study of Vintafolide (MK-8109) in Participants With Advanced Solid Tumor (MK-8109-011)	Solid Tumor	EC145	I	Terminated in 2014
NCT01953536	Safety and Efficacy Study of Vintafolide and Vintafolide Plus Paclitaxel Compared to Paclitaxel Alone in Participants With Triple Negative Breast Cancer (TNBC) (MK-8109-004)	Breast Neoplasms	EC145; Paclitaxel 80 mg/m^2^; Etarfolatide;	II	Withdrawn in 2014
			Folic acid; Premedication for Paclitaxel		
NCT01577654	Phase 2 Study of EC145 Alone Versus EC145+Docetaxel Versus Docetaxel Alone in Participants With FR(++) 2nd Line Non Small Cell Lung Cancer	Non Small Cell Lung Cancer	EC145, EC145 + Docetaxel; Docetaxel, EC20	II	Completed in 2015
NCT01170650	Study for Women With Platinum Resistant Ovarian Cancer Evaluating EC145 in Combination With Doxil®	Ovarian Cancer	EC145; Pegylated Liposomal Doxorubicin (PLD/Doxil^®^/Caelyx^®^)	III	Suspended in 2015
			placebo; EC20		
NCT00507741	Study of Vintafolide (MK-8109, EC145) in Participants With Advanced Ovarian and Endometrial Cancers (MK-8109-007, EC-FV-02)	Ovarian Cancer	EC145, Etarfolatide	II	Completed in 2015
		Endometrial Cancer			
NCT00511485	Study of Vintafolide (MK-8109, EC145) in Participants With Progressive Adenocarcinoma of the Lung (MK-8109-008, EC-FV-03)	Adenocarcinoma of the Lung	EC145, Etarfolatide	II	Completed in 2015
NCT00722592	Platinum Resistant Ovarian Cancer Evaluation of Doxil and Vintafolide (MK-8109, EC145) Combination Therapy (8109-009, EC-FV-04)	Ovarian Cancer	EC145; pegylated liposomal doxorubicin (PLD); EC20	II	Completed in 2015
NCT01688791	A Study of MK-8109 (Vintafolide) Given Alone or With Chemotherapy in Participants With Advanced Cancers (MK-8109-001)	Advanced Cancer	EC145, Carboplatin, Paclitaxel	I	Terminated in 2015
NCT01778920	Pilot and Feasibility Study of the Imaging Potential of EC17: Intraoperative Folate-fluorescein Conjugate (EC17) Lung Cancer (CA)	Lung and Pleural Malignancies Neoplasms Nodules Adenocarcinoma	EC17	I	Completed in 2016
NCT02000778	EC17 for Intraoperative Imaging in Occult Ovarian Cancer	Ovarian Cancer	EC17	I	Completed in 2018
NCT01994369	Intraoperative Imagery of Breast Cancer With Folate-FITC (EC17)	Resectable Breast Cancer	EC17	I	Completed in 2018
NCT02629549	Intraoperative Imaging of Pituitary Adenomas by OTL	Neoplasms Pituitary Neoplasms	OTL38	I	Terminated in 2018
NCT02317705	Phase 2 Study of OTL38 for Intra-operative Imaging of Folate Receptor-alpha Positive Ovarian Cancer	Ovarian Cancer	OTL38	II	Completed in 2019
NCT01999738	Folic Acid-Tubulysin Conjugate EC1456 In Patients With Advanced Solid Tumors	Solid Tumors	EC1456, EC20	I	Completed in 2019
		Non Small Cell Lung Carcinoma			
NCT03011320	An Exploratory Study of the Folic Acid-tubulysin Conjugate EC1456 in Ovarian Cancer Subjects Undergoing Surgery	Ovary Cancer	EC1456, Etarfolatide	I	Completed in 2019
NCT03180307	OTL38 for Intra-operative Imaging of Folate Receptor Positive Ovarian Cancer	Ovarian Cancer	OTL38	III	Completed in 2020
NCT02872701	OTL38 Injection for Intraoperative Imaging of Folate Receptor Positive Lung Nodules	Lung Neoplasms	OTL38	II	Completed in 2020
		Lung Cancer			
NCT02602119	Intraoperative Imaging of Pulmonary Nodules by OTL38	Neoplasms	OTL38	I	Recruiting
NCT04241315	ELUCIDATE: Enabling Lung Cancer Identification Using Folate Receptor Targeting	Lung Neoplasms	OTL38	III	Recruiting
		Lung Cancer			

EC17—folate-FITC (fluorescein isothiocyanate);EC20—etarfolatide, folate, -peptide- ^99m^technetium (Tc); EC145—vintafolide, conjugate of vinblastine monohydrazine and folic acid; EC1456—vinblastine monohydrazine and folic acid; EC0225—folate-desacetylvinblastine hydrazide or folate-mitomycin C; EC0489—folate–desacetylvinblastine hydrazide with modified linker; OTL38—folate-indole-cyanine green-like conjugate.

**Table 3:** Patented folic acid-targeted nanoparticles.

Number	Patent Title	Type of DDS
CA2487564A1	Folic acid-chitosan-DNA nanoparticles	NPs
US2010040694A1	Low-molecular weight, water-soluble chitosan nanoparticle for gene delivery with folic acid conjugated thereto as target ligand and preparation method therefor	NPs
CN102824306A	Folic acid modified chitosan coated plasmid nanoparticles and preparation method thereof	NPs
CN102961759A	Targeting gene transferring method of folic acid-functionalized PAMAM (polyamidoamine dendrimers) wrapped by gold nanoparticles	dendrimers
CN103223178A	Preparation method of folic acid modified multifunctional targeted contrast agent magnetic iron oxide/gold nanoparticles	NPs
CN103143041A	Preparation method of targeted MRI (magnetic resonance imaging) contrast medium based on folic acid modified iron oxide nanoparticles	NPs
CN103251595A	Technology for preparing folic acid-glucan-camptothecin composite nanoparticles through supercritical CO2 anti-solvent method	NPs
CN103083682A	Folic acid modified chitosan quaternary ammonium salt-taxol polymer medicine, as well as preparation method and application thereof	NPs
CN104087555A	Folic acid targeting magnetic color-developing nanoparticles and preparation method thereof	NPs
CN103933584A	Preparation method of folic acid-modified ultra-superparamagnetic iron oxide (USPIO) nanoparticles	NPs
CN103908978A	Folic acid-nano-TiO_2_ composite photocatalyst and its preparation method and use	NPs
CN103961705A	Preparation method and application of folic acid modified hollow copper sulfide/polydopamine compound	NPs
IN680DE2013A	Folic acid funcjonalized liquid crystalline nanoparticles for improved tumour delivery of anti-cancer agents	NPs
CN104436193A	Preparation method of folic acid coupled gold nano-rod/polypyrrole/ferroferric oxide multifunctional composite nano diagnosis and treatment agent	NPs
CN105396146A	Preparation method of folic-acid-modified gold nanoparticles	NPs
CN105381474A	Preparation method of folic acid modified ferriferrous oxide/gold star-shaped nanoparticles	NPs
CN105327368A	Method for preparing fluorescent silicon dioxide coated and folic acid marked gold nanoparticles	NPs
CN106110331A	Folic acid molecule targeted magnetic nano-drug and preparation method thereof	NPs
CN105920601A	Folic acid coupled targeted ferriferrous oxide/mesoporous silica/copper sulfide nano-composite particle as well as preparation method and application thereof	NPs
CN106511453A	Preparation method of nanoparticles modified by pecan kernel tannin folic acid	NPs
CN106267248A	Lipid ultrasound micro-bubble carrying folic acid modified mesoporous silicon dioxide nanoparticles and preparation method thereof	NPs
CN107970453A	Dual-targeting delivery method of pectin nanoparticles modified by folic acid	NPs
CN110652592A	Preparation method and application of folic acid-targeted dual-drug-loaded nanoparticles	NPs
CN108578427A	Folic acid modified gold nanoparticle, preparation method thereof and applications of folic acid modified gold nanoparticle in preparation of radiosensitization therapy medicines	NPs
CN108546682A	Mixed photonic crystal composite material based on folic acid modification and application	NPs
CN110123787A	Nanoparticles having paclitaxel coated with N-succinyl chitosan modified by folic acid and small molecular polypeptide and preparation method thereof	NPs
CN110501208A	Folic acid functionalized and streptavidin modified magnetic nanoparticles and preparation method and application thereof	NPs
CN111195239A	Preparation method of folic acid targeted silymarin solid lipid nanoparticles	NPs
CN111249254A	Preparation method and application of folic acid coupling albumin nanoparticles loaded with baicalin	NPs
CN111265482A	Glycyrrhetinic acid and/or folic acid ligand modified cantharidin solid lipid nanoparticle and preparation method thereof	NPs
US2020271655A1	Folic acid functionalized copper sulfide nanoparticles for the detection of ovarian cancer cells in flow	NPs
CN111035624A	Folic acid modified ABT-737 loaded mesoporous silica nanoparticles and preparation method thereof	NPs
CN110812494A	Folic acid-modified and block copolymer-wrapped gold nanoparticles and preparation method and application thereof	NPs

**Table 4:** Examples of biotinylated nanosystems developed for anti-cancer therapy.

DDS	Material	Drug	Tumour	Status	Ref.
Nanoparticles	PEG/PCL	Ptx	unspecified	In vitro—MCF-7 cells, HeLa 229 human uterine cervix adenocarcinoma cell line	[115]
Nanoparticles	Poly(D,L-lactide-co-	Dox	unspecified	In vitro—HepG2 cells, Heps murine hepatocarcinoma cell line	[120]
	glycolide)-Lecithin-				
	Polyethylene Glycol			In vivo—mice	
Nanoparticles	TPP–PEG–biotin	Dox	breast	In vitro—MCF-7 cells, HMEC normal human primary mammary epithelial cell line	[121]
	meso-				
	tetraphenylporphyrin (TPP)–PEG–biotin				
Nanoparticles	poly(ethylene glycol)-b-	Que and Dox	breast	In vitro—MCF-7 cells, MCF-7/ADR multidrug- resistant human breast cancer cell line In vivo—mice	[122]
	poly(ε-caprolactone)				
Micelles	poly(N-2-hydroxypropyl methacrylamide)-block-	Ptx	unspecified	In vitro—A549 cells, HEC293 human embryonic kidney cell line	[123]
	poly(N-2-benzoyloxypropyl methacrylamide) (p(HPMAm)-b-p(HPMAm-Bz))				
Dendrimers	poly(amidoamine) (PAMAM)	Ptx	unspecified	In vitro—A549 cells,	[124]
Dendrimers	poly(amido)amine- diethylenetriamine	Gem	unspecified	In vitro–HeLa cells,	[125]
				HaCaT cells	
Micelles	PEG-PCL	Art	breast and others	In vitro—MCF-7 cells, HFF2 normal human	[126]
				foreskin fibroblast cell line, 4T1 cells	
				In vivo—mice	
Nanoparticles	biotin-PEG-PCL	Gnb and Nar	lung	In vitro–A549 cells	[127]
				In vivo—rats	
Nanostructured lipid carriers	polyethylene glycol 2000- distearyl phosphatidyl ethanolamine	Ds	breast	In vitro—4T1 cells, L1210 murine lymphocytic leukaemia cell line	[128]
				In vivo—mice	
‘Multi-seed’ polymeric liposomes	Biotin-mPEG2000-	Asl	unspecified	In vitro—4T1 cells	[129]
	polypeptide			In vivo—mice	
Nanoparticles	chitosan	Plasmid DNA	liver	In vitro—SMMC-	[130]
				7721 human hepatocellular carcinoma cell line, LO2 normal human hepatic cell line, SW480 human	
				colon cancer cell line, H22 cells	
				In vivo—mice	
Nanotubes	Carbon nanotubes modified with	Dox	unspecified	In vitro–HeLa cells, HepG2 cells, CHO Chinese hamster ovary cell line, HEK-293	[131]
				human embryonic kidney cell line	
Nanocarriers	poly-(ethylene glycol) bis-(amine)	GA	lung and others	In vitro—A549 cells	[132]
	(BPBA)-coated reduced graphene oxide				
Nanoparticles	Biotin Decorated Gold Nanoparticles stabilized by amine terminated lipoic acid-polyethylene glycol (PEG)	copper(II) complex	unspecified	In vitro—HeLa cells,	[133]
				HaCaT cells	
				In vivo—mice	

Ptx—paclitaxel; Dox-doxorubicin; Que—quercetin; Gem- gemcitabine; Art—artemisinin; Gnb—gefitinib; Nar—naringenin; Ds—disulfiram; Asl—asulacrine; GA—gallic acid.

**Table 5:** The examples of dual-targeted nanoparticles with folic acid.

DDS	Ligand	Material	Drug	Tumour	Status	Ref.
Micelles	FA + HA	octadecyl	Ptx	breast	In vitro—MCF-7 and MCF-7/ADR cells	[155]
					In vivo—rats	
Liposomes	FA + HA	polyethylenimine	Ptx + DNA	melanoma; hepatoma	In vitro—murine melanoma cell line B16 and HepG2 cells	[156]
Liposomes	FA + Tf	DSPE-PEG2000	Dox	glioblastoma	In vitro—C6 glioma cells and bEnd3 cells	[157]
					In vivo—rats	
Liposomes	FA + mAb225	DSPE-PEG3350	Dox	unspecified	In vitro—KB cells	[158]
Liposomes	FA + TAT peptide	DSPE-PEG2000	Dox	unspecified	In vitro—KB cells	[159]
					In vivo—mice	
Liposomes	FA + glutamic hexapeptide	SPC + Cholesterol	Ptx	bone	In vitro—MDA-MB-231 cells and MCF10A cells	[160]
					In vivo—rats; mice	
Gold Nanocomposites	FA + AS1411	AuNPs	Dox	unspecified	In vitro—Hela cells	[161]
Micelles	FA + glucose	pluronic P105	Dox	glioma	In vivo—rats	[162]
Nanoparticles	FA + galactose	polyethylene glycol-dihydroartemisinin/hydroxycamptothecin	DHA	liver	In vitro—H22 cells and HepG2 cells	[163]
					In vivo—mice	
Gold Nanoclusters	FA + trastuzumab	AuNCs	-	breast	In vitro—SK-BR3 human breast cancer and normal mouse fibroblast (L929)	[164]

FA—folic acid; Tf—transferrin; HA—hyaluronic acid; mAb225—a monoclonal antibody directed against the epidermal growth factor receptors (EGFR); Ptx—paclitaxel, Dox—doxorubicin; DHA—Dihydroartemisinin; DSPE-PEG—1,2-distearoyl-sn-glycero-3-phosphoethanolamine-N-[meth-oxy(polyethyleneglycol)]; SPC—soybean phospholipids.

**Table 6:** The examples of dual-targeted nanoparticles with biotin.

DDS	Ligand	Material	Drug	Tumour	Status	Ref.
Liposomes	Bio + Glu	modified cholesterol	Ptx	breast	In vitro—4T1 cells and MCF-7 cells	[85]
					In vivo—mice	
Dendrimers	Bio + HMGB1	PAMAM	DNA	unspecified	In vitro—HeLa cells	[170]
Nanoparticles	Bio + Gal	chitosan	5-FU	liver	In vitro—SMMC-7721 cells and LO2 cells	[171]
					In vivo—mice	

Bio—biotin; Glu—glucose; Gal—galactose; HMGB1—nuclear protein—high-motility group box; 5-FU—fluorouracil; PAMAM—poly(amidoamine).

**Table 7:** Various cell lines with positive or negative biotin receptor expression.

Name of Cell Line	Origin	Folate Receptor *	Biotin Receptor *	Ref.
MCF7	human breast cancer	+	+ (+++)	[114,174,175,176,177,178,179,180]
RasV12	human breast cancer	no data	+ (++)	[114,181]
BT-20	human breast cancer	no data	+ (++)	[114,178]
LCC6-WT	human breast cancer	no data	+ (++)	[114,178]
LCC6-MDR	human breast cancer	no data	+ (+)	[114,178]
MDA-MB 231	human breast cancer	+	+ (++)	[114,176,177,178,181]
SkBr3	human breast cancer	+	+ (++)	[114,178,179,180]
MMT06056	human breast cancer	no data	+ (+++)	[114,182]
T47D	human breast cancer	+	[179]
4T1	mouse mammary carcinoma	+	+ (+++)	[182,183]
JC	mouse mammary carcinoma	+	+ (+++)	[114,119]
KB	human papilloma	+ (+++)	+	[184,185,186]
HeLa	human cervical cancer	+ (+++)	+ (+++)	[114,154,175,177,186]
KB-V1	human cervical cancer	+ (+++)	no data	[186]
OVCAR-3	human ovarian cancer	+ (+++)	+ (++)	[114,119,187]
OV2008	human ovarian cancer	+ (+++)	+ (++)	[182]
IGROV-1	human ovarian cancer	+ (+++)	no data	[186]
SKOV-3	human ovarian cancer	+ (+++)	no data	[179,180,186,188]
SKOV-3.ip	human ovarian cancer	+ (+++)	no data	[186]
A1847	human ovarian cancer	+	no data	[179]
ID8	mouse ovarian cancer	+ (+++)	+ (++)	[178,182]
PC-3	human prostate cancer	+ (+++)	+	[176,186]
Du145	human prostate cancer	+/−	+	[177,189]
PC3	human prostate cancer	no data	+	[177]
A549	human lung carcinoma	+	+ (+++)	[114,177,190,191]
M109	mouse lung carcinoma	+	+ (+++)	[182]
Colo-26	mouse colorectal	+/−	+ (+++)	[114,182]
	adenocarcinoma			
HepG2	human hepatic carcinoma	+/−	+ (+++)	[114,177,180]
Huh7	human liver cancer	no data	+	[177]
Hep3B	human liver cancer	−	+	[177]
NCI-N87	human gastric cancer	no data	+	[94,177]
AGS	human gastric cancer	no data	+	[177]
Panc-1	human pancreatic cancer	−	+	[177,182,192]
RENCA	mouse renal	+ (+)	+ (+++)	[182]
	adenocarcinoma			
RD0995	mouse renal cancer	+ (+)	+ (+++)	[182]
P815	mouse mastocytoma	+/−	+ (+++)	[182]
BW5147	mouse lymphoma	+/−	+/−	[168]
L1210FR	mouse leukaemia	+	+	[173,178]
L1219FR	mouse lymphocytic	++	+ (+++)	[114,160,178,182,193]
	leukaemia			

* If available, the affinity of binding to the biotin or folate receptors is given in parentheses.

**Table 8:** Various cell lines with negative biotin or folate receptor expression.

Name of Cell Line	Origin	Folate Receptor	Biotin Receptor	Ref.
WI38	human normal lung fibroblasts	-	-	[114,178,190,193,194,195]
LL-2	mouse Lewis lung carcinoma	-	-	[114,182,196]
HEK-293	human embryonic kidney	no data	-	[114,131,185]
NIH3T3	mouse embryonic fibroblast	no data	-	[114,194]
HCT-116	human Colon cancer	-	-	[114,182,196]
L1210	mouse lymphocytic	-	-	[114,178,193]
	leukaemia			
BW5147	mouse lymphoma T-cell	no data	-	[114,182,196]
B16-F10	mouse melanoma	-	-	[114,195]
B16	mouse melanoma	-	-	[114,182,196]

**Table 9:** The examples of nanoparticles targeted with folic acid and biotin.

DDS	Ligand	Material	Drug	Tumour	Status	Ref.
Nanoparticles	FA + BIO	Silica-coated Fe_3_O_4_	Dox	unspecified	In vitro—A549 (human epithelial lung carcinoma) and BEAS-2B (immortalized human lung epithelial) cell lines	[197]
Nanoparticles	FA + BIO	Fe_3_O_4_	-	unspecified	In vitro—E-G7 and human HeLa cells	[198]
Micelles	FA + BIO	PLA-PEG	Ptx	unspecified	In vitro—OVCAR3 (ovarian cancer cells)	[199]
Nanomicelles	FA + BIO CD44	oHA	Ica + Cur	breast	In vitro—MCF-7 cells and BCSCs cells	[200]
					In vivo—mice	
Nanorods	FA + BIO	PELA or Styrene-maleic anhydride copolymer	Dox	unspecified	In vitro—4T1 cells and RAW 246.7 macrophages	[28]
					In vivo—mice	

oHA—oligomeric hyaluronic acid; PELA—poly(ethylene glycol)-poly(DL-lactide); Ica—icariin; Cur—curcumin.

## Data Availability

Not applicable.
